This article has been retracted.

# In-depth systems biological evaluation of bovine alveolar macrophages suggests novel insights into molecular mechanisms underlying *Mycobacterium bovis* infection

**DOI:** 10.3389/fmicb.2022.1041314

**Published:** 2022-11-30

**Authors:** Aliakbar Hasankhani, Abolfazl Bahrami, Shayan Mackie, Sairan Maghsoodi, Heba Saed Kariem Alawamleh, Negin Sheybani, Farhad Safarpoor Dehkordi, Fatemeh Rajabi, Ghazaleh Javanmard, Hosein Khadem, Herman W. Barkema, Marcos De Donato

**Affiliations:** ^1^Department of Animal Science, College of Agriculture and Natural Resources, University of Tehran, Karaj, Iran; ^2^Biomedical Center for Systems Biology Science Munich, Ludwig-Maximilians-University, Munich, Germany; ^3^Faculty of Science, Earth Sciences Building, University of British Columbia, Vancouver, BC, Canada; ^4^Faculty of Paramedical Sciences, Kurdistan University of Medical Sciences, Kurdistan, Iran; ^5^Department of Basic Scientific Sciences, AL-Balqa Applied University, AL-Huson University College, AL-Huson, Jordan; ^6^Department of Animal and Poultry Science, College of Aburaihan, University of Tehran, Tehran, Iran; ^7^Halal Research Center of IRI, FDA, Tehran, Iran; ^8^Department of Food Hygiene and Quality Control, Faculty of Veterinary Medicine, University of Tehran, Tehran, Iran; ^9^Department of Agronomy and Plant Breeding, College of Agriculture and Natural Resources, University of Tehran, Karaj, Iran; ^10^Department of Production Animal Health, Faculty of Veterinary Medicine, University of Calgary, Calgary, AB, Canada; ^11^Regional Department of Bioengineering, Tecnológico de Monterrey, Monterrey, Mexico

**Keywords:** bovine tuberculosis, hub-central gene, maximal clique centrality, *Mycobacterium bovis*, RNA-seq, systems biology, weighted gene co-expression network analysis

## Abstract

**Objective:**

Bovine tuberculosis (bTB) is a chronic respiratory infectious disease of domestic livestock caused by intracellular *Mycobacterium bovis* infection, which causes ~$3 billion in annual losses to global agriculture. Providing novel tools for bTB managements requires a comprehensive understanding of the molecular regulatory mechanisms underlying the *M. bovis* infection. Nevertheless, a combination of different bioinformatics and systems biology methods was used in this study in order to clearly understand the molecular regulatory mechanisms of bTB, especially the immunomodulatory mechanisms of *M. bovis* infection.

**Methods:**

RNA-seq data were retrieved and processed from 78 (39 non-infected control vs. 39 *M. bovis*-infected samples) bovine alveolar macrophages (bAMs). Next, weighted gene co-expression network analysis (WGCNA) was performed to identify the co-expression modules in non-infected control bAMs as reference set. The WGCNA module preservation approach was then used to identify non-preserved modules between non-infected controls and *M. bovis*-infected samples (test set). Additionally, functional enrichment analysis was used to investigate the biological behavior of the non-preserved modules and to identify bTB-specific non-preserved modules. Co-expressed hub genes were identified based on module membership (MM) criteria of WGCNA in the non-preserved modules and then integrated with protein–protein interaction (PPI) networks to identify co-expressed hub genes/transcription factors (TFs) with the highest maximal clique centrality (MCC) score (hub-central genes).

**Results:**

As result, WGCNA analysis led to the identification of 21 modules in the non-infected control bAMs (reference set), among which the topological properties of 14 modules were altered in the *M. bovis*-infected bAMs (test set). Interestingly, 7 of the 14 non-preserved modules were directly related to the molecular mechanisms underlying the host immune response, immunosuppressive mechanisms of *M. bovis*, and bTB development. Moreover, among the co-expressed hub genes and TFs of the bTB-specific non-preserved modules, 260 genes/TFs had double centrality in both co-expression and PPI networks and played a crucial role in bAMs-*M. bovis* interactions. Some of these hub-central genes/TFs, including *PSMC4*, *SRC*, *BCL2L1*, *VPS11*, *MDM2*, *IRF1*, *CDKN1A*, *NLRP3*, *TLR2*, *MMP9*, *ZAP70*, *LCK*, *TNF*, *CCL4*, *MMP1*, *CTLA4*, *ITK*, *IL6*, *IL1A*, *IL1B*, *CCL20*, *CD3E*, *NFKB1*, *EDN1*, *STAT1*, *TIMP1*, *PTGS2*, *TNFAIP3*, *BIRC3*, *MAPK8*, *VEGFA*, *VPS18*, *ICAM1*, *TBK1*, *CTSS*, *IL10*, *ACAA1*, *VPS33B*, and *HIF1A*, had potential targets for inducing immunomodulatory mechanisms by *M. bovis* to evade the host defense response.

**Conclusion:**

The present study provides an in-depth insight into the molecular regulatory mechanisms behind *M. bovis* infection through biological investigation of the candidate non-preserved modules directly related to bTB development. Furthermore, several hub-central genes/TFs were identified that were significant in determining the fate of *M. bovis* infection and could be promising targets for developing novel anti-bTB therapies and diagnosis strategies.

## Introduction

Bovine tuberculosis (bTB) is domestic livestock’s infectious and chronic respiratory disease, especially in beef and dairy cattle (Brosch et al., 2002; Waters et al., 2012; Hall et al., 2021), which has paramount economic, animal welfare, and public health consequences. Despite implementing management strategies to control and eradicate it, bTB is still a major global health threat to animal populations (Vegh et al., 2015; Lu et al., 2021). Econometric analysis has ranked bTB as the fourth most important cattle disease, causing ~$3 billion in annual losses to global agriculture (Garnier et al., 2003; McLoughlin et al., 2014). bTB is caused by infection with *Mycobacterium bovis*, a pathogenic intracellular mycobacterial species belonging to *Mycobacterium tuberculosis* complex (MTBC; Smith et al., 2006; Djelouadji et al., 2011). Previous studies have shown that at the nucleotide level, *M. bovis* has a genome sequence 99.95% identical to *M. tuberculosis*, the infectious agent of human tuberculosis (TB; Garnier et al., 2003; Hall et al., 2020), and many features of *M. tuberculosis* infection in human are also characteristic of *M. bovis* infection in cattle (Pollock and Neill, 2002; Killick et al., 2014; Waters et al., 2014; Buddle et al., 2016). Therefore, as a zoonotic agent, *M. bovis* has serious implications for human health (Olea-Popelka et al., 2017; Vayr et al., 2018).

Considering the significant perturbation that occur in the normal functioning of alveolar macrophages in response to *M. bovis* infection, greater understanding the molecular regulatory mechanisms of interactions between *M. bovis* and bovine alveolar macrophages (bAMs) as well as identification of transcriptional biomarkers could be a fundamental step in the development of next-generation diagnostics and therapeutic strategies against bTB, thereby providing novel tools for disease management (Walzl et al., 2011; Nalpas et al., 2015).

The main hypothesis is that the reprogramming of bAMs by *M. bovis* occurs through extensive changes in the expression of the genes of these cells (Nalpas et al., 2015). In a previous study, Magee et al. (2014) used the RT-PCR protocol to investigate changes in gene expression in *M. bovis*-infected bAMs and reported a significant upregulation of several innate immune genes including *TLR2*, *CCL4*, *IL1B*, *IL6*, and *TNF* and a significant downregulation of *PIK3IP1* and *FOS* genes in infected samples (Magee et al., 2014). Moreover, the recent development of genome-scale high-throughput functional genomic technologies, such as gene expression microarrays and RNA sequencing (RNA-seq), which can generate a deep and global gene expression profile (Quesnel-Vallières et al., 2019), have enabled the whole-transcriptome analysis in bovine and human cells (especially macrophages) in response to *M. bovis* (Magee et al., 2012; Nalpas et al., 2013; Vegh et al., 2015; Shukla et al., 2017; Malone et al., 2018; Wiarda et al., 2020; McLoughlin et al., 2021b; Abdelaal et al., 2022) and *M. tuberculosis* (Sharma et al., 2017; Papp et al., 2018; Wang Z. et al., 2018) infection. It is worth mentioning that most of these transcriptome studies are based on differential gene expression analysis between different conditions. This method focuses only on the individual effects of genes rather than the effect of clusters of genes (Bakhtiarizadeh et al., 2020). Indeed, genes and their associated proteins interact in complex communication/biological networks (Alm and Arkin, 2003). It is expected that systematic investigation at the networks level can better and more comprehensively explain the etiology of complex diseases and identify new disease genes and drug targets more accurately (Vinayagam et al., 2016; Li M. et al., 2018).

More recently, the integration of experimental-analytical approaches with computational algorithms has been the main perspective of systems biology to understand disease biology or other complex traits (Eissing et al., 2011). Current systems biological approaches apply network theories to multi-omics data that help advance the understanding of disease (Joshi et al., 2021). Networks are computational models that organize complex biological information quantitatively (Barabási et al., 2011). One of the influential network theories to infer system-level gene–disease associations from genome-wide gene expression is the gene co-expression network approach (van Dam et al., 2017), which is based on correlation patterns among the expression of genes (Li J. et al., 2018). Gene co-expression network-based methods have been widely used to process gene expression data obtained from microarray (Wei et al., 2015; Han, 2019; Jaime-Lara et al., 2020) and RNA-seq (Wan et al., 2018; Franco et al., 2020; Kong et al., 2020) techniques in various animal and human diseases. In this regard, a well-known and helpful co-expression network-based method is weighted gene co-expression network analysis (WGCNA; Langfelder and Horvath, 2008). This method is based on expression similarities and considers differences in the response of samples at different time points by measuring the connectivity among the genes based on gene expression correlation patterns across samples and classifying highly correlated genes into specific clusters called modules (Zhang and Horvath, 2005; Langfelder and Horvath, 2008). Furthermore, the WGCNA method can identify intramodular highly connected genes (hub genes) within the modules based on the intramodular gene connectivity, which is centrally located in the module and have the most biological relationship with the relevant trait compared to other genes in that module (Langfelder and Horvath, 2008).

Systemic approaches for disease-based studies are based on the idea that disease-perturbed protein/gene regulatory networks are different from their normal conditions (Hood et al., 2004). In this regard, WGCNA has a specific network approach called module preservation analysis, which is one of the aspects of differential network analysis and is based on changes in network topological features between different conditions (healthy vs. disease; Langfelder et al., 2011). In other words, the network preservation analysis assess whether the topological properties of the modules, such as connectivity patterns and network density in a reference set (normal conditions), are preserved in a test set (disease conditions; Langfelder et al., 2011). Therefore, the presence of the topological changes in some modules (non-preserved modules) between normal and disease conditions indicates a systemic perturbation in the co-expression patterns of that modules by the disease (Hasankhani et al., 2021b). The non-preserved modules have been highlighted as key modules for investigating complex molecular mechanisms in many diseases (Mukund and Subramaniam, 2015; Riquelme Medina and Lubovac-Pilav, 2016; Bakhtiarizadeh et al., 2018; Hasankhani et al., 2021a).

In the present study, the main assumption was that the non-preserved modules could be important candidates for a better understanding of the bTB immunomodulatory mechanisms and may also contain genes that play key roles in the *M. bovis* pathogenesis. For this purpose, for the first time, we used a combination of RNA-seq data obtained from bAMs with the network preservation method of WGCNA and functional enrichment analysis to identify non-preserved modules biologically related to the molecular mechanisms behind the interactions of alveolar macrophages and *M. bovis*. Moreover, for deeper exploration, protein–protein interaction (PPI) networks derived from the co-expressed hub genes of candidate non-preserved modules were extracted to identify crucial genes and transcription factors (TFs) that had a double centrality (hub-central genes/TFs) in both co-expression and PPI networks. This study can help us to better understand of the novel molecular regulatory mechanisms underlying bTB and accelerate the discovery of sensitive genes that lead to the immunopathogenesis of *M. bovis* infection.

## Materials and methods

### Gene expression datasets

Raw RNA-seq data from alveolar macrophages of unrelated and age-matched Holstein-Friesian male calves from a TB-free herd that were challenged with *M. bovis* AF2122/97 strain *in vitro*, were obtained from the Gene Expression Omnibus (GEO) database at the National Center for Biotechnology Information (NCBI) under the accession number of GSE62506. The data included samples from 39 *M. bovis*-infected and 39 non-infected control of 10 bAMs at 2, 6, and 24 hpi and 9 bAMs at 48 hpi. An Illumina^®^ HiSeq™ 2000 was used for RNA sequencing, and a total of 1.8 billion paired-end (2 × 90 bp) reads were generated from 78 libraries. More information of preparing data can be found in the source paper (Nalpas et al., 2015).

### RNA-seq data analysis and preprocessing

To ensure the quality of the RNA-seq data, FastQC^1^ software (version 0.11.9) was used to quality control of the raw reads. Next, in order to obtain high-quality clean reads, low-quality raw reads/bases (*Q* < 20) and adapter contamination were trimmed by Trimmomatic software (version 0.39; Bolger et al., 2014) with the following parameters: ILLUMINACLIP:Adapter.fa:2:30:10, SLIDINGWINDOW:6:20, TRAILING:20, and MINLEN:60. FastQC was used again to check the quality of the clean reads and confirm improvements. Next, the paired-end clean reads were aligned to the latest bovine reference genome (ARS-UCD1.2, release-106 from Ensemble database) using Hisat2 software (version 2.2.1; Kim et al., 2019). Finally, ENSEMBL bovine GTF (release 106) and Hisat2 SAM files were used as input for the python script HTSeq-count (version 0.13.5; Anders et al., 2014) to count the uniquely mapped reads to annotated genes using intersection-strict mode. Then, all the count files were merged into a table, and a raw gene expression matrix was created that contained read counts information of all genes for all samples. In the next step, the “voom” function of the limma R package (version 3.46.0) was used for normalization of the raw gene expression matrix to log counts per million (log-CPM; Smyth, 2005; Law et al., 2014). This normalization method estimates the mean–variance relationship of the log-counts. It generates a precision weight for each observation, therefore, works better than the RNA-seq count-based methods, opening access to the RNA-seq gene expression data to computational methods (such as WGCNA) initially developed for microarrays (Law et al., 2014). Additionally, to prevent negative effects of sampling noise and unreal correlations caused by low expressed and low variance genes for the co-expression network construction, genes with expression levels ≥1 CPM in at least five samples and standard deviation >0.25 were selected for further analysis.

### Weighted gene co-expression network analysis

Based on the assumption that (1) *M. bovis* may cause systemic perturbation in the topological structure between non-infected control and *M. bovis*-infected bAMs, (2) non-preserved modules can help to better understand the molecular mechanisms of bTB, and (3) may contain important genes that lead to the development of diagnostics strategies and therapeutic methods against *M. bovis* pathogenesis, non-infected control samples (*n* = 39) were selected as a reference set for WGCNA analysis and module detection. A weighted gene co-expression network was constructed in the non-infected control samples using the WGCNA R package (version 1.70; Langfelder and Horvath, 2008) procedures in the following steps:

1. Considering the sensitivity of WGCNA to outliers, adjacency matrices of samples were constructed using the “adjacency” function of the WGCNA R package and sample network connectivity was standardized according to the distances. Samples with a standardized connectivity score < −2.5 were defined as an outlier and excluded from the downstream analysis. Afterward, the “goodSamplesGenes” function of the WGCNA R package was used to ensure the absence of samples and genes with >50% missing entries and zero variance.
2. To construct a co-expression network with a scale-free topology, *β* = 13 was calculated using the “pickSoftThreshold” function of the WGCNA R package as an acceptable soft-thresholding power β value.
3. The weighted adjacency matrix at *β* = 13 was constructed using the bi-weight mid-correlation coefficient, which is much more robust to the outliers than the Pearson correlation (Song et al., 2012), and then transformed to into the topological overlap matrix (TOM).
4. A signed weighted gene co-expression network was constructed using average linkage hierarchical clustering analysis based on the TOM dissimilarity (1-TOM), and modules with different sizes were detected through a dynamic hybrid tree cutting algorithm.
5. Finally, modules with highly similar expression profiles were identified and then merged based on the correlation between the module eigengenes (the first principal component of the gene expression profile for a given module).

All the above steps were performed using automatic, one-step network construction and module detection function “blockwiseModules” of the WGCNA R package with the following major parameters: networkType = “signed,” TOMType = “signed,” corType “bicor,” power = 13, maxBlockSize = 16,000, reassignThreshold = 0, mergeCutHeight = 0.25, and minModuleSize 30.

### Module preservation analysis

Network preservation analysis was performed using a permutation test based on 200 random permutations *via* “modulePreservation” function of the WGCNA R package. This network-based approach examines whether the mean connection strength among all genes in a module (known as network density) and the sum of the connection strengths for a gene with other network genes (known as connectivity) are preserved between non-infected control bAMs (*n* = 39) as a reference set and *M. bovis*-infected bAMs (*n* = 39) as a test set through two composite module preservation statics including Z_summary_ and medianRank (Langfelder et al., 2011). To get an accurate result of testing the preservation level between the respective conditions, especially when modules are compared with different sizes, the Z_summary_ statistic, which is highly dependent on the module size and increases with increasing module size, should be combined with the medianRank statistic, which is module-size independent (Langfelder et al., 2011). Overall, higher Z_summary_ values and lower medianRnak values indicates a high level of preservation between different conditions, so modules with Z_summary_ > 10 or medianRank <8 are considered highly-preserved (Langfelder et al., 2011). Therefore, in the current study, modules with Z_summary_ ≤ 10 or medianRank ≥8 were defined as non-preserved between non-infected control and *M. bovis*-infected samples.

### Functional enrichment analysis of the non-preserved modules and TFs prediction

To investigate and interpret the biological behavior of non-preserved modules and to identify bTB-specific non-preserved modules, the co-expressed genes in each non-preserved module were analyzed using the Enrichr^2^ online tool based on the Gene ontology (GO) terms for biological process and Kyoto Encyclopedia of Genes and Genomes (KEGG) pathway enrichment (Chen et al., 2013). A significant threshold for functional terms was defined as an adjusted *p*-value < 0.05 (corrected by the Benjamini–Hochberg method). Additionally, a set of bovine TFs extracted from the AnimalTFDB3.0^3^ database was used to identify co-regulated TFs that played a crucial immunoregulatory role in the non-preserved modules (Hu et al., 2018).

### Identification of hub-central genes in the bTB-specific non-preserved modules

In the co-expression modules, highly connected intramodular genes, also known as hub genes, which have the highest degree of connection compared to other genes in that module, are expected to play important roles in the complex biological mechanisms of that module (Bi et al., 2015; Das et al., 2017). The central role of intramodular hub genes in candidate modules has led them to be used as potential novel biomarkers to accelerate the development of the next-generation diagnostics and therapeutic strategies against various diseases (Li S. et al., 2017; Wang L.-X. et al., 2018; Miao et al., 2019). In this regard, multiple steps were performed to identify genes with double centrality (hub-central) in the candidate non-preserved modules associated with *M. bovis* infection.

1. Module memberships (MM) or eigengene-based connectivity *k_ME_* criterion, which interprets the relationship between modules and genes (Langfelder and Horvath, 2008), was calculated through the correlation between the gene expression profile and the module eigengenes by WGCNA R package. Taken together, co-expressed genes with values of *k_ME_* ≥ 0.7 were defined as highly connected intramodular hub genes in the non-preserved modules.
2. In order to explore network density and protein interactions, the co-expressed hub genes of the bTB-specific non-preserved modules were subjected to PPI network construction using Search Tool for the Retrieval of Interacting Genes (STRING) database^4^ with medium stringency options (Szklarczyk et al., 2018).
3. Maximal clique centrality (MCC) is one of the novel local-based topological algorithms for node centrality in a network that has better performance than other topological algorithms for identifying the PPI networks hub genes (Chin et al., 2014) and has been proposed to increase the sensitivity and specificity for discovering featured nodes (Chin et al., 2014; Li and Xu, 2019). For this purpose, co-expressed hub genes-based PPI networks of each candidate non-preserved module were inputted into Cytoscape^5^ software (version 3.7.1) and interpreted with the cytoHubba plugin (version 0.1; Chin et al., 2014) based on the MCC algorithm to identify co-expressed intramodular hub genes with the highest MCC score (hub-central genes).
4. Next, the top 50 genes in co-expressed hub genes-based PPI networks of candidate non-preserved modules with a size of ≥350 and the top 20 genes in co-expressed hub genes-based PPI networks of candidate non-preserved modules with a size of ≤200 in terms of MCC score were considered as hub-central genes. Besides, co-expressed hub genes-based PPI networks of the bTB-related non-preserved modules were visualized using Cytoscape software (version 3.7.1; Cline et al., 2007).

### Validation of RNA-Seq results using quantitative real-time PCR

To validate the reproducibility of RNA-seq data, five DEGs including *BCL2L1*, *MMP1*, *EDN1*, *MAPK8*, and *CTSS* were selected for analysis by qRT-PCR. The same RNAs extracted from bovine alveolar at each non-infected control vs. *Mycobacterium bovis*-infected animals were used for qRT-PCR validation. Quantitative reverse-transcription-PCR was carried out according to the manufacturer specifications for reference to SYBR® Premix Ex TaqTM. SYBR Green PCR cycling was denatured using a program of 95°C for 10 s, 35 cycles of 95°C for 5 s, and 60°C for 40 s, and performed on an ABI 7500 instrument (United States). The specificity of each PCR product was confirmed by melting curve analysis. All qRT-PCR assays were performed in triplicate reactions. The housekeeping genes RPL19 and *GAPDH* were used as the internal control genes. The expression levels of target mRNAs were obtained based on RNAs extracted from bovine alveolar and were shown to be normalized to *GAPDH*. Forward and reverse primer sequences and accession numbers of selected genes are given in Supplementary Table S1.

## Results

### RNA-seq data summary

Overall details of RNA-seq data analysis and weighted gene co-expression network construction steps are schematically presented in Figure 1. Totally 1,769,182,596 RNA-seq raw reads of 39 non-infected control bAMs and 39 *M. bovis*-infected bAMs (an average of 23 million paired-end reads per sample) were retrieved and processed. After quality control and trimming, a total of 1,751,490,782 high quality clean reads were obtained. On average, 85% of the clean reads were uniquely aligned to the bovine reference genome, and the overall mapping rate was 94%. complete details of RNA-seq data and preprocessing are provided in Supplementary Table S2. In order to minimize the sampling noise, different parameters were applied and a total of 10,563 genes were kept for co-expression network analysis. The final normalized gene expression profile is available in Supplementary Table S3.

**Figure 1:** Schematic pipeline of RNA-seq data analysis and weighted gene co-expression network construction steps.

### Weighted gene co-expression network construction and module detection

To better understand the molecular mechanisms underlying bTB, the normalized and filtered gene expression matrix obtained from RNA-seq data analysis were combined with WGCNA approaches. Based on the details obtained from the adjacency matrices of samples, two samples, GSM1528042 and GSM1528044, had a standardized connectivity score < −2.5 and were excluded as an outlier (Figure 2; Supplementary Table S4). The weighted gene co-expression network was constructed based on the TOM dissimilarity at β = 13, which represents a scale free topology fitting index (*R*^2^) ≥ 0.80 (Figure 3; Supplementary Table S5), and a total of 21 modules (excluding 576 uncorrelated genes in gray module) in different sizes were identified in the non-infected control samples as the reference set through hierarchical clustering analysis and dynamic hybrid tree cutting algorithms, and each module was labeled with a specific color by WGCNA method. The identified co-expression modules as branches of the gene hierarchical clustering dendrogram are shown in Figure 4. The average size of each module was 476 genes and turquoise module with a size of 2,521 genes and darkred module with a size of 40 genes were identified as the largest and smallest module, respectively. Complete information of the identified modules is presented in Supplementary Table S6.

**Figure 2:** Sample clustering to detect outliers in the non-infected controls bAMs as reference set for module detection. Based on the adjacency matrices of samples, two samples including GSM1528042 and GSM1528044 had a standardized connectivity score < −2.5 and were excluded as outlier.

**Figure 3:** Network topology analysis. **(A)** Scale-free topology fitting index (*R*^2^) (*y*-axis) and **(B)** mean connectivity (*y*-axis) for different soft-threshold powers (*β*) (*x*-axis). The weighted gene co-expression network was constructed at *β* = 13, which represents a scale free topology fitting index (*R*^2^) ≥ 0.80.

**Figure 4:** Gene hierarchical clustering dendrogram of detected modules across all samples. A total of 21 modules in different sizes were identified based on the TOM dissimilarity (1-TOM) in the non-infected control bAM samples as reference set through hierarchical clustering analysis and dynamic hybrid tree cutting algorithms. The *x*-axis represents the genes and the *y*-axis represents the co-expression distance. The branches indicate the modules, and each module was labeled with a unique color. The gray module including 576 genes indicate uncorrelated genes.

### Network preservation analysis

Module preservation analysis was performed to investigate changes in network properties between non-infected control samples (*n* = 39) as a reference set and *M. bovis*-infected samples (*n* = 39) as a test set. The results showed that among 21 modules identified in non-infected control samples, the network density and connectivity patterns of 14 modules were altered in *M. bovis*-infected samples, making them key candidates for studying the biological mechanisms of bTB disease. Accordingly, the topological structure of 7 modules, including lightyellow, midnightblue, gray60, greenyellow, royalblue, lightcyan, and black, was highly preserved between the respective conditions (Figure 5). Among the highly preserved modules, lightyellow and midnightblue modules had the highest degree of topological preservation between non-infected control and *M. bovis*-infected samples. On the other hand, in agreement with our primary assumption, 14 modules, including brown, purple, darkred, tan, yellow, salmon, green, cyan, magenta, pink, turquoise, lightgreen, red, and blue were systematically perturbed by *M. bovis* infection (Figure 5). Moreover, the blue module with a size of 1805 co-expressed genes had the most significant alteration in network characteristics in response to *M. bovis* infection. Further details of the module preservation analysis are provided in Supplementary Table S7.

**Figure 5:** Module preservation analysis. **(A)** The medianRank preservation statistics. The *y*-axis represents medianRank values for different modules and the *x*-axis represents module size. Each point indicates a module labeled by a unique color. The blue dashed line represents the medianRank threshold. **(B)** The Z_summary_ preservation statistics. The *y*-axis represents Z_summary_ values for different modules and the *x*-axis represents module size. Each point indicates a module labeled by a unique color. The red dashed line represents the Z_summary_ threshold. Modules with Z_summary_ ≤ 10 or medianRank ≥8 were considered as non-preserved between non-infected control and *Mycobacterium bovis*-infected conditions.

### Functional enrichment analysis of the non-preserved modules

Functional enrichment analysis was performed to investigate biological processes and KEGG pathways to detect the specific molecular mechanisms of the non-preserved modules and the functional differentiation between them. In total, 642 biological processes were significantly enriched in 12 non-preserved modules. No biological processes were significantly enriched in the other two non-preserved modules, the darkred and lightgreen modules. Furthermore, the KEGG pathway enrichment analysis showed that 194 pathways were significantly enriched in 11 non-preserved modules, including blue, brown, green, red, pink, purple, salmon, tan, turquoise, yellow, and magenta. Interestingly, the most non-preserved module between non-infected control and *M. bovis*-infected bAMs, the blue module, had the highest enrichment rate in the KEGG pathways and biological processes (234 and 50 biological processes and KEGG pathways, respectively). The top 10 significant biological processes and KEGG pathway GO terms of the non-preserved modules are shown in Figures 6, 7, respectively. Based on the interpretation of the functional enrichment results, out of 14 non-preserved modules, 7 non-preserved modules, including blue, brown, green, pink, salmon, tan, and turquoise, were directly related to the host immune response, immunomodulatory mechanisms of *M. bovis* infection, and bTB development. Some of these critical pathways and processes were included “Apoptosis,” “Ferroptosis,” “regulation of cell cycle phase transition (GO:1901987),” “negative regulation of mitotic cell cycle phase transition (GO:1901991),” “negative regulation of cell cycle G2/M phase transition (GO:1902750),” “positive regulation of Wnt signaling pathway (GO:0030177),” “JAK–STAT signaling pathway,” “PI3K-Akt signaling pathway,” “negative regulation of programmed cell death (GO:0043069),” “negative regulation of apoptotic process (GO:0043066),” “T cell receptor signaling pathway,” “regulation of T cell activation (GO:0050863),” “Th17 cell differentiation,” “Th1 and Th2 cell differentiation,” “Natural killer cell mediated cytotoxicity,” “gamma-delta T cell activation (GO:0046629),” “positive regulation of interferon-gamma production (GO:0032729),” “B cell receptor signaling pathway (GO:0050853),” “Toll-like receptor signaling pathway,” “C-type lectin receptor signaling pathway,” “NOD-like receptor signaling pathway,” “RIG-I-like receptor signaling pathway,” “Cytosolic DNA-sensing pathway,” “IL-17 signaling pathway,” “NF-kappa B signaling pathway,” “MAPK signaling pathway,” “negative regulation of type I interferon production (GO:0032480),” “Necroptosis,” “Fatty acid degradation,” “fatty acid catabolic process (GO:0009062),” “fatty acid beta-oxidation (GO:0006635),” “regulation of lipid metabolic process (GO:0019216),” “fatty acid oxidation (GO:0019395),” “cholesterol metabolic process (GO:0008203),” “secondary alcohol biosynthetic process (GO:1902653),” “fatty acid beta-oxidation using acyl-CoA oxidase (GO:0033540),” “regulation of cholesterol biosynthetic process (GO:0045540),” “cellular amino acid catabolic process (GO:0009063),” “Tryptophan metabolism,” “Valine, leucine and isoleucine degradation,” “Glycine, serine and threonine metabolism,” “Autophagy,” “regulation of macroautophagy (GO:0016241),” and “regulation of autophagy (GO:0010506).” Complete information from the results of the functional enrichment analysis of non-preserved modules is presented in Supplementary Table S8.

**Figure 6:** Dot plot of functional enrichment analysis. The top 10 significant biological process GO terms of the non-preserved modules. The *y*-axis represents significant enriched GO terms and the *x*-axis represents module name. Color and size of each point represent adjusted *p*-value and number of genes for each term, respectively.

**Figure 7:** Dot plot of functional enrichment analysis. The top 10 significant KEGG pathway GO terms of the non-preserved modules. The *y*-axis represents significant enriched GO terms and the *x*-axis represents module name. Color and size of each point represent adjusted *p*-value and number of genes for each term, respectively.

### Identification of TFs, hub TFs, hub genes, and hub-central genes in the candidate non-preserved modules

In this study, module preservation and functional enrichment analysis identified 7 candidate non-preserved modules, including blue, brown, green, pink, salmon, tan, and turquoise, that were biologically related to bTB pathogenesis. To identify crucial intramodular hub genes that played a central role in the biological function of these modules, the MM criterion was calculated by the WGCNA R package. A total of 3,653 co-expressed hub genes were identified with *k_ME_* ≥ 0.7 in all non-preserved modules (Supplementary Table S9). Taken together, a total of 725, 382, 170, 222, 140, 134, and 938 highly connected hub genes were screened in the blue, brown, green, pink, salmon, tan, and turquoise candidate non-preserved modules, respectively. Additionally, important TFs that regulated the transcription of co-expressed genes in the non-preserved modules were extracted based on the bovine transcriptional regulatory factors of AnimalTFDB3.0 database, and a total of 491 TFs were identified in all non-preserved modules (Supplementary Table S10). Besides, among the co-expressed hub genes identified in the non-preserved modules, a total of 22, 12, 8, 26, 6, 14, and 29 TFs (hub TFs) were detected in the blue, brown, green, pink, salmon, tan, and turquoise bTB-specific non-preserved modules, respectively (Supplementary Table S11). Intriguingly, the co-expressed intramodular hub genes of the 7 candidate non-preserved modules were densely connected in the PPI networks based on the STRING database information, indicating close biological relationships between proteins encoded by these genes. Eventually, 260 hub-central genes were identified in the bTB-specific non-preserved modules, which have a double centrality in both PPI and co-expression networks and could be key candidates for better understanding the complex etiology of bTB, development of diagnostics and potential therapeutic targets for *M. bovis* infection (Table 1; Supplementary Table S12). Moreover, the co-expressed hub genes-based PPI networks of the bTB-specific modules are displayed in Figure 8.

**Table 1:** List of the hub-central genes/TFs identified in the bTB-specific non-preserved modules.

Module						
Blue	Brown	Green	Pink	Salmon	Tan	Turquoise
*PSMA3*	*SRC*	*CD3E*	*TNF*	*SRSF3*	*NFKB1* ^*^	*EHHADH*
*PSMD14*	*MMP9*	*CD4*	*IL6*	*SRSF2*	*NFKB2* ^*^	*HADH*
*PSMC5*	*VCL*	*ZAP70*	*IL1B*	*TRA2B*	*CD40*	*PCCA*
*PSMC1*	*ITGB1*	*CD247*	*GRO1*	*SNRPB2*	*IKBKE*	*ALDH6A1*
*PSMD8*	*ITGB3*	*LCK*	*IL1A*	*PRPF38A*	*TRAF2*	*PCCB*
*PSMD2*	*RHOC*	*CD3D*	*NFKBIA*	*TRA2A*	*LYN*	*HIBADH*
*PSMA4*	*TENC1*	*CD3G*	*TNFAIP3*	*SRSF7*	*PRKCD*	*ALDH7A1*
*PSMC4*	*YES1*	*ITK*	*TLR2*	*SNRPC*	*CTNNB1*	*ALDH2*
*PSMD12*	*CCND1*	*PIK3CD*	*PTGS2*	*MX1*	*MAP2K1*	*ABAT*
*PSMC3*	*FLT1*	*BOLA-DRA*	*CCL4*	*MX2*	*STAT6* ^*^	*ALDH9A1*
*PSMD6*	*STAT1* ^*^	*LA-DQB*	*CCL20*	*RNPS1*	*MAPK7*	*ECHDC1*
*PSMA2*	*LPP*	*BOLA-DRB3*	*ICAM1*	*DHX58*	*IL23R*	*DBT*
*PSMB2*	*BCL2L1*	*PRKCQ*	*CXCL3*	*USP18*	*BRD2* ^*^	*ACSS1*
*PSMB7*	*CDKN1A*	*IL2RB*	*IRF1* ^*^	*IFIT2*	*PSEN1*	*ACSS2*
*PSMA1*	*CSF2*	*IL2RA*	*NFKBIZ*	*DDX46*	*TNIP1*	*ALDH3A2*
*PSMA5*	*HSPG2*	*CD2*	*VEGFA*	*TRAF1*	*CD274*	*ECHS1*
*PSMD1*	*FLNA*	*LOC100300510*	*TBK1*	*IL10*	*NAPB*	*ACAA1*
*PSMA6*	*CCND2*	*MATK*	*MAP3K8*	*RIPK2*	*SNAP29*	*GCDH*
*PSMB3*	*EZR*	*BLK*	*IRAK2*	*CASP4*	*TNFSF13B*	*MCCC1*
*PSMD7*	*PLAUR*	*CD52*	*CCL8*	*NAIP*	*ESRRA* ^*^	*OXCT1*
*PSMB6*	*PDGFB*	*–*	*DUSP1*	*–*	*–*	*CAT*
*PSMD13*	*CSF1*	*–*	*ATF3* ^*^	*–*	*–*	*MUT*
*PSMB4*	*MDM2*	*–*	*EDN1*	*–*	*–*	*ACAD10*
*PSMD4*	*SDC1*	*–*	*NLRP3*	*–*	*–*	*SCP2*
*VCP*	*ITGB8*	*–*	*ISG15*	*–*	*–*	*C1QA*
*PSMD11*	*CTLA4*	*–*	*NFKBIE*	*–*	*–*	*C1QC*
*ADRM1*	*VLDLR*	*–*	*HIF1A* ^*^	*–*	*–*	*CTSS*
*PSMD3*	*CDC25A*	*–*	*MAPK8*	*–*	*–*	*ACSF2*
*PSMA7*	*ITGAD*	*–*	*ZC3H12A*	*–*	*–*	*C1QB*
*PSMB10*	*CSF2RB*	*–*	*BIRC3*	*–*	*–*	*C3AR1*
*PSMB5*	*HBEGF*	*–*	*TNFAIP6*	*–*	*–*	*CRYL1*
*PSME1*	*TIMP1*	*–*	*RND1*	*–*	*–*	*PECR*
*PSMD5*	*PARVA*	*–*	*JUNB* ^*^	*–*	*–*	*LAP3*
*PSME2*	*MMP1*	*–*	*FOSL1* ^*^	*–*	*–*	*LY86*
*USP14*	*CD69*	*–*	*IER3*	*–*	*–*	*FCGR3A*
*COPS5*	*PTPN22*	*–*	*MEFV*	*–*	*–*	*VSIG4*
*TXNL1*	*RRAS2*	*–*	*FOSB* ^*^	*–*	*–*	*DERA*
*PSMG2*	*CD38*	*–*	*PTX3*	*–*	*–*	*ADH5*
*CCT5*	*YWHAZ*	*–*	*UTP15*	*–*	*–*	*BDH2*
*UFD1L*	*IL7R*	*–*	*BRIX1*	*–*	*–*	*LY9*
*UBQLN1*	*LIMK1*	*–*	*RRP12*	*–*	*–*	*FYB*
*EIF3I*	*DSTN*	*–*	*KRR1*	*–*	*–*	*PEPD*
*PES1*	*IDO1*	*–*	*PAK1IP1*	*–*	*–*	*CTSD*
*EBNA1BP2*	*CCL22*	*–*	*DDX5*	*–*	*–*	*LAPTM5*
*NOC2L*	*IL13RA1*	*–*	*DDX59*	*–*	*–*	*VPS18*
*BYSL*	*GPC1*	*–*	*RSAD2*	*–*	*–*	*VPS11*
*PNO1*	*WEE1*	*–*	*UBA7*	*–*	*–*	*FCGR1A*
*RBM28*	*ENAH*	*–*	*SNAI1* ^*^	*–*	*–*	*STX10*
*PWP1*	*IL1RN*	*–*	*EIF3CL*	*–*	*–*	*VPS33B*
*DDX47*	*DCSTAMP*	*–*	*JAG1*	*–*	*–*	*TREM2*

* The asterisks represent the bovine hub-central TFs.

**Figure 8:** PPI network derived from co-expressed hub genes of the **(A)** green, **(B)** turquoise, **(C)** blue, **(D)** salmon, **(E)** tan, **(F)** pink, and **(G)** brown modules. Large circles and orange round rectangles represent hub-central genes and TFs, respectively.

### Analysis of expression based on qRT-PCR data

To assess the accuracy and the reliability of differential expression genes identified by RNA-seq, five DEGs from non-infected control vs. *Mycobacterium bovis*-infected samples were selected to perform qRT-PCR tests. The expression results for five genes were assessed using RNA-seq and qRT-PCR and are shown in Figure 9. As can be observed, the expression patterns of five genes showed a general agreement between the two technologies.

**Figure 9:** Differentially expressed genes were selected from transcriptome comparison combinations at different non-infected control vs. *M. bovis*-infected samples. The black-filled columns represent the relative mRNA expression levels obtained by qRT-PCR, which were normalized by *GAPDH*; **(A)** *BCL2L1* gene expression, **(B)** *MMP1* gene, **(C)** *EDN1* gene expression, **(D)** *MAPK8* gene expression, **(E)** *CTSS* gene expression, The gray columns show the log2 (FC) value obtained by RNA-seq.

## Discussion

bTB is a severe infectious disease caused by infection with *M. bovis* and inflicts irreparable economic losses on the dairy and beef cattle industry (Middleton et al., 2021). However, an insufficient understanding of the molecular regulatory mechanisms behind bTB has been one of the main reasons for the limitation of various techniques to control or eradication this disorder in recent decades (Schiller et al., 2010; Fang et al., 2020). Combining high-throughput technologies with novel computational systems biology approaches provide new opportunities to better understand the molecular mechanisms underlying various diseases (Sharifi et al., 2019). Therefore, in this study, a combination of RNA-seq data with module preservation analysis (a network-based method of WGCNA) was used to obtain a comprehensive insight into the complex mechanisms involved in the interactions of bovine host and *M. bovis* infection. Briefly, a signed weighted gene co-expression network was constructed and a total of 21 modules were identified in the non-infected control bAM samples as a reference set for network preservation analysis. Generally, signed networks provide a better understanding of the biological mechanisms behind traits/diseases at the systematic level and differentiate the potential functions of the modules better and more accurately (Mason et al., 2009). In agreement with the main hypothesis of this study, *M. bovis* infection in bAMs was able to change the network characteristics of 67% of the identified modules (14 out of 21) compared to the non-infected control bAMs. Then, functional enrichment analysis based on the biological processes and KEGG pathways showed that among the 14 non-preserved modules, 7 non-preserved modules, including blue, brown, green, pink, salmon, tan, and turquoise were directly involved in host-pathogen interactions and could be important candidates for studying pathogenic mechanisms of bTB as in previous similar studies, these candidate non-preserved modules were successfully used as key modules to describe the complex etiology of several bovine diseases, such as bovine mastitis (Bakhtiarizadeh et al., 2020), bovine respiratory disease (BRD; Hasankhani et al., 2021b), bovine endometritis (Sheybani et al., 2021), and Johne’s disease (Heidari et al., 2021). It should be noted that loss of connection or alteration of the connectivity patterns and network density in the non-preserved modules can be attributed to the abnormal expression of several genes in *M. bovis*-infected conditions, which can be key factors in the development of bTB. Therefore, several steps were performed to identify these key dysregulated genes, including identification of intramodular hub genes in the non-preserved modules, integration of co-expressed hub genes with PPI networks, and identification of the hub-central genes in the bTB-specific co-expressed hub genes-based PPI networks through MCC topological algorithm. Noteworthy, in parallel with the current study, the MCC algorithm has been used as an objective criterion for measuring node centrality and identifying important genes/proteins in candidate networks in disease-based system biology studies (Bai et al., 2020; Yang et al., 2020; Ma et al., 2021; Wang Y. et al., 2021). Finally, a total of 260 hub-central genes were found in the 7 bTB-specific non-preserved modules that these genes were hubs in their co-expression networks and also played a central role in the respective co-expressed hub genes-based PPI networks (so-called double centrality) which were as critical targets in related to the promotion of the bTB establishment.

Co-expressed genes in the blue module showed high enrichment in KEGG pathways such as “Apoptosis,” “Ferroptosis,” “Tuberculosis,” and “Proteasome,” as well as biological processes including “regulation of cell cycle phase transition (GO:1901987),” “negative regulation of mitotic cell cycle phase transition (GO:1901991),” “negative regulation of cell cycle G2/M phase transition (GO:1902750),” “positive regulation of Wnt signaling pathway (GO:0030177),” and “Fc-gamma receptor signaling pathway involved in phagocytosis (GO:0038096).” Apoptosis is a programmed cell death that is one of the possible consequences of host-pathogen interaction in mycobacterial infections (Behar et al., 2011; Mohareer et al., 2018). Apoptosis is a potential defense mechanism against intracellular pathogens. There is growing evidence that apoptosis of infected macrophages can limit the proliferation and growth of intracellular mycobacteria and subsequently reduce mycobacterial viability (Allen et al., 2001; Benítez-Guzmán et al., 2018; Abdalla et al., 2020). Several previous studies have shown that *M. tuberculosis* infection in humans (Keane et al., 1997; PLACIDO et al., 1997) and murine (Rojas et al., 1998) and *M. bovis* infection in cattle (Gutiérrez-Pabello et al., 2002; Vega-Manriquez et al., 2007) induce apoptosis in macrophages. Additionally, it has been highlighted that the reduction of *M. bovis* growth in bovine macrophages has a positive and significant correlation with the induction of apoptosis in infected macrophages (Denis et al., 2007). Therefore, it has been suggested that the induction of apoptosis is closely linked to the emergence of macrophage resistance to *M. bovis* replication (Denis et al., 2005). On the other hand, apoptosis may act as a double-edged sword, so uncontrolled apoptosis of macrophages and T cells during infection may play an important role in the formation of tuberculous lesions (Fayyazi et al., 2000; Cassidy, 2006).

During *M. bovis* infection, various types of cell death may be induced, among which apoptosis and autophagy restricts bacterial growth and facilitates host defense mechanisms, while ferroptosis and necroptosis are beneficial for pathogen growth and transmission (Chai et al., 2020). Ferroptosis is a new type of iron-dependent programmed necrotic cell death caused by intracellular iron accumulation and lipid peroxidation, leading to oxidative stress and cell death (Chen et al., 2021b). Significantly, infections with MTBC agents such as *M. bovis* and *M. tuberculosis* induce the appearance of necrotic lesions (Cassidy, 2006; Harper et al., 2011; Roy et al., 2019). Indeed, it has been hypothesized that ferroptosis plays an essential role in the pathogenesis of MTBC infectious agents through (1) iron accumulation which is an essential component for successful infection of various infectious bacilli causing TB, and (2) induction of necrosis (Meunier and Neyrolles, 2019). Consistent with our results, these findings suggest the importance of ferroptosis during infection with infectious agents of MTBC, which could be a promising target for the control and treatment of *M. bovis* and *M. tuberculosis* infections.

Bacterial pathogens use a variety of strategies to manipulate host cell function to their advantage, thereby evading the host’s immune responses and prolonging infection (Nougayrède et al., 2005). One of these immunomodulatory mechanisms for escaping the immune responses is to induce the host cell cycle arrest. In this regard, an in-depth transcriptomic effort showed that *M. tuberculosis* could arrest the cell cycle of macrophages in mice, potentially modulating the host immune response and enhancing long-term persistence (Cumming et al., 2017). Therefore, treatment strategies based on interference with pathogen-host cell cycle interactions can be effective approaches for chemotherapeutic intervention to prevent long-term infection of intracellular bacilli (Cumming et al., 2017).

The Wnt signaling pathway is an important ancient molecular cascade that plays a key role in many developmental processes and the maintenance of adult tissue homeostasis by interfering with processes such as regulating cell proliferation, migration, preservation of adult stem cells, differentiation, apoptosis, the immune response (Blumenthal et al., 2006; Schaale et al., 2011), and genetic stability (Kahn, 2014; Duan and Bonewald, 2016). Additionally, it has recently been reported that dysregulation in the Wnt signaling are linked to the pathogenesis of lung diseases, especially lung cancer, pulmonary fibrosis, and pulmonary arterial hypertension (Königshoff and Eickelberg, 2010).

Interestingly, several hub-central genes of the blue module, such as *PSMB3*, *PSMA3*, *PSMA4*, *PSMB4* (Seto et al., 2020), *PSMA5* (Widdison et al., 2011), *PSMD6*, *PSMB6*, *PSMD8* (Zhao et al., 2022), *PSME2* (Maji et al., 2015), *PSME1* (Bell et al., 2017), and *PSMC4* (Shi et al., 2021) involved in the proteasome pathway, played important roles in the pathogenesis of *M. bovis* and *M. tuberculosis*. For instance, the *PSMB3*, *PSMA3*, *PSMA4*, and *PSMB4* hub-central genes are associated with mycobacterial granulomatous lesions (Seto et al., 2020). Moreover, integrated bioinformatic research identified the *PSMC4* hub-central gene as one of the important biomarkers for tuberculous pleurisy (Shi et al., 2021). Among the other hub-central genes in the blue module, we also identified two genes, including *COPS5* (Meenu et al., 2016; Sambarey et al., 2017) and *UBQLN1* (Sakowski et al., 2015; Franco et al., 2017), that were associated with the host immune responses, leading to restriction of mycobacterial growth/replication and clearance of intracellular *M. bovis*, respectively.

Functional enrichment analysis revealed that the brown module was significantly enriched in several immune/pathogenic-related pathways such as “JAK–STAT signaling pathway,” “PI3K-Akt signaling pathway,” “negative regulation of programmed cell death (GO:0043069),” and “negative regulation of apoptotic process (GO:0043066).” The Janus kinase/signal transducers and activators of transcription (JAK–STAT) pathway is one of a handful of pleiotropic cascades that is the major signal transducer for a wide range of cytokines and growth factors (Vainchenker and Constantinescu, 2013). The JAK–STAT signaling pathway begins with the extracellular binding of cytokines as well as IFNs to their respective receptors, which leads to receptor oligomerization and then accelerates JAKs trans-activation. Following the activation of JAKs, the cytoplasmic tails of the receptors are phosphorylated, which puts JAKs and STATs in spatial proximity. Then, JAKs mediate tyrosine-phosphorylation (p-Tyr) of STATs, which results in STAT dimerization, nuclear translocation, DNA binding and, finally, regulation of gene transcription (Villarino et al., 2017; Xin et al., 2020). Pathogenic mycobacteria can interfere with the JAK–STAT signaling pathway and attenuate the cytokine-induce immune response. Previous studies have discovered one of the immunosuppression and survival strategies of pathogenic mycobacteria such as *M. bovis* (Imai et al., 2003; Fang et al., 2020), *M. tuberculosis* (Manca et al., 2005), and *Mycobacterium avium* subsp. *paratuberculosis* (MAP; Arsenault et al., 2014) in macrophages is the blockade of the JAK–STAT signaling pathway by inducing this pathway inhibitor’s expression.

It is well known that the phosphatidylinositol 3-kinase (PI3K)/protein kinase B (AKT) signaling pathway plays a vital role in cell growth, metabolism, differentiation, apoptosis, and autophagy (Yu and Cui, 2016; Zhang et al., 2017). As discussed in the blue module, apoptosis of macrophages infected with intracellular bacilli such as *M. bovis* and *M. tuberculosis* actively destroys infected host cells and their contents, including intracellular mycobacteria, thereby limiting mycobacterial growth and proliferation (Behar et al., 2011; Nalpas et al., 2015). In contrast, research has shown that one of the major mechanisms of escaping the host immune response and increasing mycobacterial survival is macrophage apoptosis subversion by *M. bovis* and *M. tuberculosis* (Keane et al., 2000; Behar et al., 2011; Abdalla et al., 2020; Fang et al., 2020). Interestingly, activation of the PI3K-Akt signaling pathway during mycobacterial infection directly modulates the apoptosis of host cells (Gong et al., 2020). Additionally, Hussain et al. (2019a) observed that *M. bovis* disrupted autophagosome assembly by activating the PI3K-Akt signaling pathway, thereby modulating autophagy and thus preventing intracellular pathogen degradation (Hussain et al., 2019a). Furthermore, it has recently been revealed that infectious agents of MTBC, through some of its proteins, inhibits the production of proinflammatory cytokines and reduces antigen-presenting cell (APC) function in mouse macrophages *via* the activation of PI3K-Akt signaling pathway (Liu et al., 2016). Nevertheless, these results suggest that the PI3K-Akt signaling pathway plays important roles in the pathogenesis of *M. bovis* and other MTBC infectious agents and could be considered in future research as a promising target for bTB control. Moreover, in agreement with the biological performance of the brown module, other immune/pathogenic-related processes of the brown module including “Cytokine-cytokine receptor interaction,” “cytokine-mediated signaling pathway (GO:0019221),” and “Focal adhesion” have been observed in similar network-based TB studies (Lin et al., 2019; Li L. et al., 2020; Alam et al., 2022; Liang et al., 2022).

Additionally, in terms of the hub-central genes identified in the brown module, several hub-central genes such as *SRC* (Chandra et al., 2016), *ITGB3* (Chen et al., 2021a), *BCL2L1* (Sharma et al., 2016), *CDKN1A* (Silva et al., 2021), *MDM2* (Shariq et al., 2021), and *MMP1* (Villarreal-Ramos et al., 2018) have been reported as key factors in the immunomodulatory mechanisms of MTBC agents such as *M. bovis*. It is well known that phagocytosis is an effective immune response process in killing intracellular mycobacteria, while mycobacteria prevent phagocytosis by host cells to maintain survival within macrophages (Fang et al., 2020). Interestingly, research has reported that *M. tuberculosis* infection leads to upregulation of the *SRC* hub-central gene, which directly inhibits phagosome-lysosome fusion and plays an effective role in maintaining mycobacterial survival within macrophages (Lechartier et al., 2014). In this regard, it has been highlighted that inhibition of *SRC* promotes phagosome acidification and xenophagy flux in macrophages, and *SRC* inhibitors have a substantial potential for developing anti-TB drugs (Chandra et al., 2016). Moreover, another study showed that, unlike the *SRC* hub-central gene, upregulation of the *ITGB3* hub-central gene could overcome the inhibition of phagosome maturation due to mycobacterial infection, and activation of *ITGB3* could facilitate *M. tuberculosis* clearance *in vivo* (Chen et al., 2021a). The *BCL2L1* hub-central gene is an important anti-apoptotic factor that has shown a significant upregulation in response to *M. bovis* and *M. tuberculosis* infections, and it has been suggested that this hub-central gene plays a central role in the pathogenic mechanisms of infectious bacilli by inhibiting apoptosis (Xaus et al., 1999; Nalpas et al., 2015; Silva et al., 2021). In addition to *BCL2L1*, the *CDKN1A* hub-central gene encodes the p21 protein, a member of the Cip/Kip family, whose high levels are associated with pulmonary sarcoidosis and, as an inhibitor of apoptosis, facilitate the formation and maturation of TB granulomas (Xaus et al., 1999, 2003; Silva et al., 2021). Furthermore, the *M. tuberculosis* RipA (a peptidoglycan hydrolase) suppresses the caspase-mediated apoptosis pathway by activation the *MDM2* hub-central gene and continues its survival in the infected host (Shariq et al., 2021). Interestingly, the results of previous studies suggest that the *MDM2* hub-central gene showed higher levels of expression in response to infection with virulent strains of *M. bovis* (AF2122/97) than attenuated strains (G18) and with greater inhibition of apoptosis in macrophages infected with AF2122/97 played a crucial role in the development of bTB (Jensen et al., 2018). The *MMP1* is another hub-central gene whose gene products are key to collagen degradation and alveolar destruction (Salgame, 2011). Indeed, it has been reported that *M. tuberculosis*, as well as *M. bovis*, selectively upregulated *MMP1* gene expression, which leads to tissue destruction in TB and immunopathology of the lungs (Elkington et al., 2011; Parasa et al., 2017; Villarreal-Ramos et al., 2018).

Other hub-central gene of the brown module, including *CSF1* (Chatterjee et al., 2021), *PLAUR* (McLoughlin et al., 2021b), *ITGB1* (Yang et al., 2017), *CCND1* (Koo et al., 2012; Looney et al., 2021), *CSF2* (Marsay et al., 2013; Shukla et al., 2017; Abdelaal et al., 2022), *CTLA4* (Zhang et al., 2021), *FLNA* (Xu et al., 2015), *CCND2* (Lavalett et al., 2017), *WEE1* (Jayaswal et al., 2010), *MMP9* (Blanco et al., 2012; McLoughlin et al., 2014), *CDC25A* (Shapira et al., 2020), *CSF2RB* (Benmerzoug et al., 2018), *TIMP1* (Sun et al., 2020), *CD69* (Li et al., 2011; Chen et al., 2020), *PTPN22* (Boechat et al., 2013), *CD38* (Silveira-Mattos et al., 2019), *IL7R* (Jenum et al., 2016; Alsulaimany et al., 2022), *IL1RN* (Alcaraz-López et al., 2020), and *IDO1* (Weiner et al., 2012; Gautam et al., 2018) were also involved in host-pathogen interactions as well as suppression of host immune response. For example, the *CTLA4* hub-central gene encodes an inhibitor of T cell-mediated response (Schneider et al., 2006), and the upregulation of this gene in response to *M. bovis* infection may reflect a mechanism of immunomodulation used by *M. bovis* to subvert a host T-cell response (Killick et al., 2011). The *WEE1* hub-central gene plays an important role in combating the progression of infection and intracellular survival of *M. tuberculosis*. It has been reported that knocking down the *WEE1* gene leads to a significant increase in Mycobacterium levels in host macrophages (Jayaswal et al., 2010). It has also been reported that the *MMP9* and *TIMP1* hub-central genes were highly correlated with TB development (Klepp et al., 2019), and have been suggested as valuable diagnostic biomarkers for TB (Xu et al., 2015; Sun et al., 2020) and bTB (Blanco et al., 2012). Moreover, the *IL1RN* hub-central gene has been suggested as a promising candidate biomarker for natural resistance to bTB in Holstein-Friesian cattle (Alcaraz-López et al., 2020).

In the brown module, we also identified *STAT1* hub-central TF, a pivotal component of the JAK–STAT signaling pathway and a signal transducer and transcription activator that mediates cellular responses to IFNs, cytokines, and growth factors (Hall et al., 2020). Interestingly, *M. bovis* counteracts the immune response by suppressing *STAT1* expression and exacerbates its pathogenesis in the host cells (Chen J. et al., 2021). Studies in patients with active TB have shown that *STAT1* activation was impaired in host macrophages (Esquivel-Solís et al., 2009). Additionally, it has been proved that *M. tuberculosis* EspB protein suppresses IFN-γ-induced autophagy in murine macrophages by inhibiting IFN-γ-activated *STAT1* phosphorylation (Huang and Bao, 2016). Most importantly, unphosphorylated *STAT1* inhibits apoptosis in *M. tuberculosis*-infected macrophages (Yao et al., 2017). Surprisingly, *STAT1* leads to the expression of inducible nitric oxide (NO) synthase and subsequently releases NO at sufficient concentrations for mycobactericidal. Thus, it can be concluded that *M. bovis* inhibits the mycobactericidal mechanism of NO by inhibiting *STAT1* phosphorylation (Sharma et al., 2007). Therefore, these findings demonstrate the importance of *STAT1* hub-central TF in the host immune response during mycobacterial infection, which could be a key target for counteracting *M. bovis* immunosuppressive strategies and developing a treatment for bTB in the future.

Functional terms such as “T cell receptor signaling pathway,” “regulation of T cell activation (GO:0050863),” “Th17 cell differentiation,” “Th1 and Th2 cell differentiation,” “Natural killer cell mediated cytotoxicity,” “gamma-delta T cell activation (GO:0046629),” “positive regulation of interferon-gamma production (GO:0032729),” and “B cell receptor signaling pathway (GO:0050853)” showed that the green module is closely related to the cell-mediated and humoral immunity. There is considerable evidence from various *in vitro* and *in vivo* studies that indicate the central role of T-cell subtypes (γδ, CD4 and CD8 T-cells) in host defense against mycobacterial pathogens, including *M. bovis* (POLLOCK et al., 1996; Cassidy et al., 2001), as demonstrated in the absence of T-cells, TB susceptibility increases (Mogues et al., 2001; Moguche et al., 2017). Furthermore, progressive impairment of the *M. tuberculosis*-specific T-cell responses with increasing mycobacterial load and subsequent recovery of responses during the treatment period indicates an inverse relationship between T-cell activation and disease severity of TB (Day et al., 2011). The production of IFN-γ by CD4 T-cells to activate the bactericidal mechanisms of infected macrophages is an essential process for host defense against bTB and TB (Flynn et al., 1993; Vordermeier et al., 2002; Gallegos et al., 2011; Cooper and Torrado, 2012). It has also been reported that γδ T-cells may significantly limit *M. bovis* infection by producing IFN-γ (Kennedy et al., 2002). On the other hand, it has been observed that cytotoxic T-cells inhibit the growth of intracellular mycobacteria by special lysis of *M. bovis*-infected macrophages (Skinner et al., 2003). In particular, the design of new vaccines and vaccination strategies based on CD8 T-cell responses has been proposed (Kaufmann et al., 1999). According to previous research, in agreement with the adaptive immune response of the green module, following the initiation of a cell-mediated immune response, the initiation of humoral immunity specially B-cell-dependent signals, such as “B cell receptor signaling pathway” during *M. bovis* infection, may be involved in the mycobactericidal response in bTB (Pollock et al., 2006; Aranday-Cortes et al., 2012).

Interestingly, most of the hub-central genes in the green module, including *CD3E* (Mair et al., 2021), *ZAP70* (Samten et al., 2009), *CD4* (Boggiatto et al., 2021), *IL2RA* (Lu et al., 2011), *CD247*, *LCK*, *CD3D*, *CD3G*, *PRKCQ* (McLoughlin et al., 2021a), and *ITK* (Huang et al., 2020), were closely related to T-cell activation and the host immune response to infection with MTBC intracellular pathogens. The *CD3E* hub-central gene is an essential core for T-cell activation (Mair et al., 2021) and plays a crucial role in the immune response against TB (Gebremicael et al., 2019). Based on the results of previous research, an intense decrease in the expression of *CD3E* in patients with active TB and then an increase in the expression of this gene during the treatment period exhibited that this gene has a negative correlation with the progression of mycobacterial infection (Jenum et al., 2016; Gebremicael et al., 2018). In addition to *CD3E*, the *ZAP70* and *LCK* hub-central genes are key components of T-cell activation and signaling, and there is growing evidence that intracellular mycobacteria such as *M. bovis* and *M. tuberculosis* interfere with the function of host T-cells by downregulating the phosphorylation of these genes (Mahon et al., 2012; Sande et al., 2016). *ITK* is a tyrosine kinase that regulates T-cells development and function. Indeed, *ITK* deficiency and alternation in T-cell receptor/ITK signaling impairs early protection against *M. tuberculosis* in human lungs (Huang et al., 2020). Therefore, enhancing of ITK signaling has been introduced as an alternative strategy to target infection with highly virulent strains of *M. tuberculosis* (Huang et al., 2020). Remarkably, several hub-central genes of the green module, including *ITK*, *CD2*, *CD247*, *ZAP70*, *CD3D*, and *CD3E*, were identified as potential therapeutic targets for pulmonary TB by a computational drug-ability effort (Alsulaimany et al., 2022).

The results of the functional enrichment analysis suggested that co-regulated genes of the pink module were highly enriched in the host innate immune response and inflammatory mechanisms such as “Toll-like receptor signaling pathway,” “C-type lectin receptor signaling pathway,” “NOD-like receptor signaling pathway,” “RIG-I-like receptor signaling pathway,” “Cytosolic DNA-sensing pathway,” “IL-17 signaling pathway,” “NF-kappa B signaling pathway,” “MAPK signaling pathway,” “negative regulation of type I interferon production (GO:0032480)” and “Necroptosis.” Pathogen-associated molecular pattern molecules (PAMPs) are essential components derived from microorganisms that are critical to the survival and function of microorganisms (Akira et al., 2006; Tang et al., 2012). Indeed, recognition of mycobacterial PAMPs by PRRs of innate immune cells, such as macrophages, activates a cascade of downstream signaling, which ultimately leads to the activation of the nuclear factor kappa B (NF-κB) and mitogen-activated protein kinase (MAPK) signaling pathways (Trinchieri and Sher, 2007; Gong et al., 2020). Finally, activation of the NF-κB and MAPK downstream signaling pathways leads to the host inflammatory response through the production of proinflammatory cytokines and chemokines such as *IL6*, *IL1B*, *TNF*, *IL18*, and *IL8*, which in addition to inducing an innate immune response, regulate subsequent adaptive immune response (Means et al., 2000; Mahla et al., 2013; Thakur et al., 2018). However, various reports suggest that *M. tuberculosis* and *M. bovis* modulates proinflammatory cytokine production *via* the NF-κB and MAPK signaling inhibition in favor of their survival and thus suppresses the innate immune response (Pathak et al., 2007; Wang et al., 2015; Liu et al., 2016; Ha et al., 2020; Lu et al., 2020). On the other hand, activation of NF-κB and MAPK signaling pathways can also play an important role in TB immunopathology (Bai et al., 2013). Moreover, overactivity of the NF-κB and IL-17 signaling pathways in response to mycobacterial infection leads to the induction of pyroptosis which is a highly inflammatory form of lytic programmed cell death, thereby facilitating the spread of mycobacteria to neighboring cells (Beckwith et al., 2020) as well as severe TB sepsis (Li L.-L. et al., 2020). This finding indicates the importance of the inflammatory pathways as key targets for inducing different immunosuppressive strategies by MTBC pathogens.

Overall, PRRs are divided into two main categories: (1) membrane-bound PRRs including Toll-like receptors (TLRs) and C-type lectin receptors (CLRs); and (2) cytoplasmic PRRs including NOD-like receptors (NLRs) and RIG-I-like receptors (RLRs; Killick et al., 2013). Several previous transcriptomic studies have highlighted that *M. bovis* infection induces the toll-like receptor signaling pathway in bovine macrophages (Lin et al., 2015; Ma et al., 2016; Shukla et al., 2018). Nevertheless, in addition to the important role that TLRs play in initiating an innate immune response and enhancing adaptive immunity, mycobacterial activation of TLR signaling may act as an escape mechanism from host defense (Netea et al., 2004). Therefore, it has been recommended that modulation of TLR signaling could affect ability of invading mycobacteria such as *M. bovis* to destroy and escape the host response (Krutzik and Modlin, 2004).

Other factors, including NLRs and RLRs, interact with the activation of inflammatory responses and thus help induce an innate immune response (Zitvogel et al., 2012). The NLR family is a group of cytoplasmic receptors involved in inflammation and immunity by interfering with the secretion of several cytokines and playing a considerable role in mycobacterial-host interactions (Pahari et al., 2017). Based on the results of time series studies, activation of the NOD-like receptor signaling pathway in the early stages of infection with virulent strains of *M. bovis* in bovine macrophages indicates a key role of these pathways to induce a robust macrophage response to infection with mycobacterial pathogens (Jensen et al., 2018). Additionally, several studies have highlighted the central role of NLRs in various aspects of the host immunity, including resistance to *M. tuberculosis* infection (Divangahi et al., 2008) and restriction of intracellular *M. tuberculosis* growth by inducing autophagy in infected human alveolar macrophages (Juárez et al., 2012), optimal production of proinflammatory cytokines (Brooks et al., 2011), and enhancing NO production (Landes et al., 2015). RLRs are a group of RNA helicases that play an important role in the detection of viral RNA in the host cytoplasm (Killick et al., 2013). Generally, RLR signaling is involved in the production of type I IFNs and antiviral proteins by activating downstream transcription factors (Loo and Gale, 2011). It has been made clear that the expression of several genes commonly associated with the detection of viral PAMPs, such as viral RNA, is manipulated during the *M. bovis* challenge *in vitro*, suggesting that the RIG-I-like receptor signaling pathway may be involved in the mycobacterial infections (Magee et al., 2012). Furthermore, based on the functional biological process term “negative regulation of type I interferon production (GO:0032480)” of the pink module, we hypothesized that *M. bovis* may modulate the production of type I IFNs. This hypothesis is supported by previous transcriptomic studies that reported that *M. bovis* and *M. tuberculosis* actively reduced the production of type I IFNs in bovine, human, and murine macrophages and dendritic cells to increase their survival and immune evasion (Simmons et al., 2010; Nalpas et al., 2015; Banks et al., 2019).

As mentioned, mycobacterial pathogens such as *M. bovis* and *M. tuberculosis* kills infected macrophages by inhibiting apoptosis and autophagy and promoting necrosis. However, the induction of necrosis is associated with the formation of granuloma, which is the hallmark of TB infection (Butler et al., 2012). Necroptosis is a prototype of programmed necrosis death, also known as inflammatory programmed cell death, and is considered as the link between cell death and inflammation (Mohareer et al., 2018). In other words, necroptosis exacerbates the host inflammatory response to infection and therefore contributes significantly to tissue damage (Tripathi et al., 2018). Besides, previous reports have shown that intracellular *M. tuberculosis* induces necroptosis in myeloid lineage cells such as monocytes and macrophages, leading to (1) exacerbation of necrosis and (2) impaired trained immunity, thereby facilitates mycobacterial escape and dissemination (Khan et al., 2020). Interestingly, a recent study suggested that inhibition of necroptosis may improve the health status of TB patients and enhance antibacterial TB chemotherapy (Pajuelo et al., 2020).

Several inflammation-related genes, including *TLR2* (Meade et al., 2007), *NLRP3* (Malone et al., 2018), *CCL4* (Widdison et al., 2008), *IL1A*, *IL1B*, *TNF* (Salgame, 2005), and *IL6* (Magee et al., 2012) had double centrality in both co-expression network and co-expressed hub gene-based PPI network of the pink module and played a central role in the interactions between bAMs and *M. bovis*. One of the essential mechanisms of host defense against intracellular pathogens is innate immunity, which is highly dependent on the behavior of inflammatory molecules. Thus, proinflammatory cytokines such as *TNF*, *IL6*, *IL1A*, and *IL1B* are core component of the host’s innate immune response against invading *M. bovis* (Salgame, 2005). Increased expression of *TNF*, *IL6*, *IL1B*, and *IL1A* hub-central genes in bovine monocyte-derived macrophages (bMDMs) following *in vitro* stimulation with *M. bovis* in a 48 h time series indicates their important role in the early-stage of infection (Wang et al., 2011; Magee et al., 2014; Sabio y García et al., 2020). Conversely, suppression *TNF* and *IL6* gene expression to counteract the host immune response is a key feature of late-stage of *M. bovis* infection (MacHugh et al., 2009). Interestingly, various reports have demonstrated that the use of *TNF* antagonists and inhibitors increases (1) TB susceptibility, (2) reactivation of *M. bovis* and *M. tuberculosis*, (3) and risk of TB mortality in humans and cattle (Ehlers, 2003; Nager et al., 2009; Xie et al., 2014; Arbués et al., 2020). Moreover, blocking or inactivating the *TNF* hub-central gene leads to *M. bovis* escaping from the TNF-induced apoptosis of host macrophages (Piercy et al., 2007). These findings indicate a key role of *TNF* hub-central gene in preventing TB or bTB reactivation and limiting the pathogenic response of the host.

Another study showed that in addition to *TNF*, polymorphisms of another cytokine genes such as *IL1B* and *IL6* were associated with latent TB infection and pulmonary TB (Wu et al., 2018, 2019). Besides, the use of an additional readout system, such as *IL1B*, has been suggested to increase the sensitivity of IFN-γ release assay (IGRA) test for the detection of *M. bovis* infection in cattle (Jones et al., 2010). Additionally, *TNF* and *IL1A* hub-central genes have been identified as promising biomarkers for the development of bTB diagnosis strategies (Sánchez-Soto et al., 2017; Palmer et al., 2020). *TLR2* hub-central gene is a major component of the TLR family and plays an important role in recognizing mycobacterial PAMPs and activating the innate immune response (Nalpas et al., 2015). *TLR2* signaling acts as a potential defense system against *M. bovis* infection because the host innate immune response to MTBC infectious agents is mainly mediated by *TLR2* in macrophages and leads to the activation of macrophages in the early stage of infection (Krutzik and Modlin, 2004). Moreover, activation of *TLR2* also induces apoptosis as a direct bactericidal effect in infected macrophages and suppresses the proliferation of intracellular mycobacteria (Gerold et al., 2007). Interestingly, as a survival strategy and subversion mechanism of the host immune response, *M. tuberculosis* suppresses *TLR2* through several of its components, such as LprE lipoprotein and PPE51 protein, and subsequently inhibits *TLR2*-dependent autophagy and cathelicidin (Padhi et al., 2019; Strong et al., 2022). The use of *TLR2* agonists has also been highlighted as an effective tool for optimizing vaccination strategies to protect cows against bTB (Wedlock et al., 2008).

However, in addition to the key role that these inflammation-related hub-central genes play in the host-pathogen interactions, they can act as a double-edged sword and play an effective immunopathological role during *M. tuberculosis* and *M. bovis* infection. For instance, overexpression of the *IL6* in *M. tuberculosis* or *M. bovis*-infected macrophages can inhibit the macrophage response to IFN-γ (Nagabhushanam et al., 2003) and suppress the T-cell response (Magee et al., 2012). Significantly, pathogenic mycobacteria can interfere with host defense mechanisms through TLRs. As mentioned earlier, long-term stimulation of *TLR2* in *M. tuberculosis*-infected macrophages suppresses the IFN-γ response (Gehring et al., 2003) and inhibits antigen presentation in infected macrophages (Noss et al., 2001). *NLRP3* inflammasome is an important member of the intracellular NLR family, and previous bioinformatics research has reported a rapid increase in the expression of this gene in response to virulent strains of *M. bovis* infection in macrophages (Zhou et al., 2016). Indeed, *NLRP3* inflammasome activates *CASP1*, leading to the release of *IL1B*, which in turn leads to pyroptosis in *M. tuberculosis*-infected macrophages, resulting in severe ultrastructural disruptions and spread of the pathogen in the host cells (Beckwith et al., 2020; Kanipe and Palmer, 2020). Additionally, *NLRP3* activation is directly related to necrotic death triggered by *M. tuberculosis* (Wong and Jacobs, 2011). *CCL4* is a proinflammatory and chemotactic beta chemokine that has been shown to play an important role in the *respiratory syncytial virus* (RSV), *bovine immune deficiency virus*, and *M. bovis* infections (Widdison and Coffey, 2011). Previous reports indicate an increase in the *CCL4* expression levels in response to *M. bovis* (Nalpas et al., 2013), and growing evidence suggests a direct positive correlation between *CCL4* plasma levels and bTB-induced lung lesions (Widdison et al., 2009).

Other hub-central genes of the pink module were included *CCL8* (Rusk et al., 2017), *CCL20* (Malone et al., 2018), *CXCL3* (Zhang et al., 2019), DUSP1 (Abo-Kadoum et al., 2021), *EDN1* (Lin et al., 2015), *ICAM1* (Li P. et al., 2017), *IER3* (Widdison et al., 2011), *ISG15* (Kimmey et al., 2017), *MAP3K8* (Naeem et al., 2021), *NFKBIA* (Tsai et al., 2009), *NFKBIZ* (Dong et al., 2022), *PTGS2* (Xiong et al., 2018), *PTX3* (Wang et al., 2013), *RSAD2* (Andreu et al., 2017), *TBK1* (Wang J. et al., 2018), *MAPK8* (Gautam et al., 2014), *BIRC3* (MacHugh et al., 2012), *TNFAIP3* (Hall et al., 2020), *TNFAIP6* (Lin et al., 2015), and *VEDFA* (Ndlovu and Marakalala, 2016), and the intracellular pathogen of MTBC such as *M. bovis*, could induce various strategies to escape the host immune response by activating or suppressing these genes. According to the literature reports on models of *M. tuberculosis* and *M. bovis* infection, some of these molecular mechanisms that contribute to the TB pathogenesis include the following:

1. Overexpression of *CCL20* in response to *M. tuberculosis* infection reduces ROS production and subsequently inhibits ROS-dependent apoptosis (Rivero-Lezcano et al., 2010).
2. A 700-fold increase in expression of the *EDN1* hub-central gene has been reported in *M. bovis*-infected cows. The *EDN1* gene encodes the ET-1 protein, which leads to increased pulmonary hypertension, delayed T-cell response, and inhibition of the migration of antigen-presenting cells (Lin et al., 2015).
3. *Mycobacterium tuberculosis* inhibits P53-dependent apoptosis by activating *PTGS2* (Dutta et al., 2012).
4. The *ICAM1*, *PTGS2*, *CCL20*, and *IL6* hub-central genes showed a close relationship with the development of pulmonary TB and had the potential to use biomarkers for TB (Sun et al., 2020).
5. A recent study using *in vitro* and *ex vivo* approaches discovered that miR-199a expression increased significantly in response to *M. bovis* infection. Subsequently, miR-199a suppresses cellular autophagy, apoptosis and modulates the production of type I IFNs by directly targeting the *TBK1* hub-central gene (a major regulator of autophagy), thereby accelerating intracellular growth and survival of *M. bovis* (Wang J. et al., 2018).
6. *Mycobacterium bovis* and *M. tuberculosis* inhibit host cell apoptosis by increasing expression in anti-apoptotic factors such as *BIRC3* (Killick et al., 2014) and decreasing expression in pro-apoptotic factors such as *MAPK8* (Gautam et al., 2014). Moreover, interventional methods to activate *MAPK8* have been proposed as a potential therapeutic strategy to increase apoptosis of infected cells and destruction of intracellular mycobacteria (Alam et al., 2021).
7. Increased expression of *VEGFA* in patients with active TB leads to the development of TB granuloma associated angiogenesis (Ndlovu and Marakalala, 2016).
8. The *TNFAIP3* hub-central gene is a central regulator of immunopathology because it is a key player in the negative feedback regulation of the NF-κB signaling pathway (Vereecke et al., 2009), and increased of *TNFAIP3* expression levels in *M. bovis*-infected animals modulates the host immune response and decreases proinflammatory cytokines (especially *TNF*) by inhibition NF-κB signaling, thereby leads to progression of *M. bovis* infection (Kumar et al., 2015).

Several hub-central TFs, including *ATF3* (Chen Y. et al., 2021), *FOSB* (Green et al., 2010), *HIF1A* (Li F. et al., 2020), and *IRF1* (Pathak et al., 2007) were also identified that played a key immunoregulatory role in the biological behavior of the pink module. For example, *HIF1A* hub-central TF is a master transcriptional regulator and an important factors in regulating gene expression in response to hypoxia (Cimmino et al., 2019). *HIF1A* TF plays a key role in combating *M. bovis* infection, as previous studies have shown that interfering *HIF1A* with siRNA defected the capacity of phagocytosis, ROS generation, and glucose metabolism (Li F. et al., 2020). On the other hand, *HIF1A* is also effective in host-directed anti-TB immunometabolism processes (Shi et al., 2015). *IRF1* hub-central TF is the first member of the interferon-regulatory transcription factor (IRF) family to be initially introduced as an IFN-beta (a type I IFN) transcription activator (Yarilina et al., 2008). In this regard, as mentioned earlier, *M. tuberculosis* through some of its proteins, inhibits the activation of IFN-associated TFs, such as *IRF1*, and modulates the production of type I IFNs (Pathak et al., 2007).

In addition to the pink module, we identified several critical functional terms related to inflammation and immune response, such as “NF-kappa B signaling pathway,” “TNF signaling pathway,” and “B cell receptor signaling pathway” in the tan module, as well as terms such as “cytokine-mediated signaling pathway (GO:0019221),” “negative regulation of programmed cell death (GO:0043069),” “toll-like receptor 2 signaling pathway (GO:0034134),” and “negative regulation of epithelial cell apoptotic process (GO:1904036)” in the salmon module. Moreover, several hub-central genes/TFs of the tan module such as *CD40* (Khan et al., 2016), *CD274* (Petrilli et al., 2020), *CTNNB1* (Subuddhi et al., 2020), *IKBKE* (Killick et al., 2014), *IL23R* (Jiang et al., 2015), *MAPK7* (María Irene et al., 2021), *TRAF2* (Killick et al., 2014), *NFKB1* (Meade et al., 2007), *NFKB2* (Magee et al., 2012), and *STAT6* (Cronan et al., 2021), as well as hub-central genes of the salmon module, such as *CASP4* (Malone et al., 2018), *DHX58* (Nalpas et al., 2015), *IL10* (Wang et al., 2011), *MX1*, *MX2*, *IFIT2* (Yi et al., 2021), *RIPK2* (Widdison et al., 2011), *TRAF1* (Li H. et al., 2017), and *USP18* (Carranza et al., 2020), have been reported to be involved in the host immunity and *M. bovis* pathogenesis. The *NFKB1* hub-central TF is a major mediator of the proinflammatory immune response that stimulates the transcription of proinflammatory cytokines and chemokines and has shown a significant reduction in the response to *M. bovis* infection (Meade et al., 2007). Interestingly, several previous studies have highlighted that a decrease in *NFKB1* expression in response to *M. tuberculosis* and *M. bovis* infection is directly related to suppression of the host innate immune signaling as well as prevention of phagosome maturation in the chronic stages of bTB and TB (MacHugh et al., 2009; Alam et al., 2019). Furthermore, *IL10* is an anti-inflammatory cytokine that has been upregulated in response to *M. bovis* infected bovine macrophages (Wang et al., 2011). Indeed, several previous researches suggests that *M. bovis*, as well as *M. tuberculosis* induces various immunomodulatory mechanisms, including inhibition of phagosome-lysosome fusion and, thus prevention of phagosome maturation (O'Leary et al., 2011), suppression of the production of IFN-γ, NO, and proinflammatory cytokines such as *TNF*, *IL6* and *IL1B* (Jensen et al., 2019), in infected macrophages by upregulating *IL10* expression levels (Sheridan et al., 2017). Therefore, direct gene repression of *IL10* during *M. tuberculosis* infection has been proposed as a novel solution to improve macrophage bactericidal functions and *M. tuberculosis* clearance (Chandra et al., 2013).

Significant functional terms such as “Fatty acid degradation,” “fatty acid catabolic process (GO:0009062),” “fatty acid beta-oxidation (GO:0006635),” “regulation of lipid metabolic process (GO:0019216),” “fatty acid oxidation (GO:0019395),” “cholesterol metabolic process (GO:0008203),” “secondary alcohol biosynthetic process (GO:1902653),” “fatty acid beta-oxidation using acyl-CoA oxidase (GO:0033540),” “regulation of cholesterol biosynthetic process (GO:0045540),” “cellular amino acid catabolic process (GO:0009063),” “Tryptophan metabolism,” “Valine, leucine and isoleucine degradation,” and “Glycine, serine and threonine metabolism” in the turquoise module have supported the hypothesis that host metabolic processes are reprogrammed by intracellular mycobacteria such as *M. bovis* as well as *M. tuberculosis* (Lee et al., 2013).

During mycobacterial infections, especially the virulent strains of *M. tuberculosis* and *M. bovis*, extraction and utilization of host nutrients, especially fatty acids and cholesterol (preferably) for the survival and viability of mycobacteria is essential for all pathogenic activities by these pathogens (Lee et al., 2013). Several studies using *M. tuberculosis* infection models have been reported that this pathogen has a unique ability to assimilate and utilize host-derived lipids, especially fatty acids and cholesterol, which catabolized as important carbon sources to fuel central metabolic pathways to facilitate the mycobacterial growth and persistence (Cole et al., 1998; Russell et al., 2009; Wilburn et al., 2018). In addition to carbon sources, mycobacterial pathogens can provide the required nitrogen sources through the metabolism of amino acids in the host (Gouzy et al., 2014). For example, host serine (Ser) biosynthesis is one of the most important processes to provide the nitrogen sources needed for *M. tuberculosis* survival (Borah et al., 2019). Additionally, tryptophan (Trp) metabolism plays a vital role in the growth and activation of MTBC infectious agents (Qualls and Murray, 2016), so there is growing evidence that during *M. tuberculosis* infection, activated macrophages try to limit growth of intracellular pathogen through Trp starvation. However, in return, *M. tuberculosis* induces Trp biosynthesis in the host to counteract this auxotroph threat (Wang X. et al., 2021).

Important hub-central genes of the turquoise module were included *ACAA1* (Behera et al., 2022), *ACAD10* (Nalpas et al., 2015), *ACSS2* (Koo et al., 2012), *ALDH2* (Park et al., 2014), *ALDH9A1* (Aiyaz et al., 2014), *C1QA*, *C1QB*, *CIQC* (Cai et al., 2014), *C3AR1* (Zhang et al., 2019), *ECHS1* (Bell et al., 2017), *EHHADH* (Aiyaz et al., 2014), *FCGRA1* (Jenum et al., 2016), *LAPTM5* (Kang et al., 2011), *PCCA*, *PCCB* (Katiyar et al., 2018), *PEPD* (White et al., 2010), *TREM2* (Iizasa et al., 2021), *VPS11*, *VPS18* (Chandra et al., 2015), and *VPS33B* (Mascarello et al., 2010), which were involved in the host immune response and bAMs-*M. bovis* interactions. For instance, *ACAA1* is one of the core component of fatty acid metabolic process which encodes a hallmark enzyme of fatty acid β-oxidation, and it has been reported that *M. tuberculosis* increases the rate of fatty acid β-oxidation for its survival by enhancing the expression of this gene (Behera et al., 2022). Besides, *ALDH2* has a protective effect on TB by interfering with alcohol metabolism (Park et al., 2014). C1q is a 460 kDa protein consisting of 18 polypeptide chains (6A, 6B, and 6C) whose main function is to initiate complement activation. It has been observed that high levels of C1q subtype proteins such as *C1QA*, *C1QB*, and *C1QC* are strongly associated with active TB and disease severity (Lubbers et al., 2018). In addition, *C1QC* has been introduced as a potential biomarker for active TB diagnosis (Cai et al., 2014). Moreover, the *PEPD* hub-central gene is essential in facilitating mycobacterial adaptation (White et al., 2010) and is directly associated with cavity formation in patients with pulmonary TB (Wang et al., 2014). *VPS33B* is a subset of the class C vacuolar protein sorting complex (Vps-C) that acts as the core of membrane fusion and protein sorting (HOPS) and regulates membrane trafficking throughout the endocytic pathway (Wong et al., 2013). Intriguingly, *M. tuberculosis* protein tyrosine phosphatase A (PtpA) dephosphorylates and inactivates *VPS33B*, thereby shutting down the membrane fusion machinery in the host macrophages (Wong et al., 2011). As a result, inactivation of *VPS33B* directly blocks phagosome-lysosome fusion and prevents phagosome acidification (Bach et al., 2008; Chen, 2015).

We also identified autophagy related pathways such as “Autophagy,” “regulation of macroautophagy (GO:0016241),” and “regulation of autophagy (GO:0010506)” in the turquoise module. During the autophagy, cytoplasmic packages, including damaged organelles, misfolded proteins, and intracellular pathogens, are enclosed in a double-membrane vesicle called autophagosome and after fusion with a lysosome (autophagosome maturation), an autolysosome is formed which decomposes its contents (Hasankhani et al., 2021a). Numerous studies have reported that autophagy is a direct mechanism for killing intracellular *M. tuberculosis* and *M. bovis*, and protecting the host against TB (Ní Cheallaigh et al., 2011; Castillo et al., 2012; Songane et al., 2012; Hussain et al., 2019b). Conversely, as discussed, intracellular tubercle bacilli escape autophagy using specific immunosuppressive strategies. In this regard, we identified several hub-central genes, including *CTSS*, *VPS11*, *VPS18*, and *VPS33B* in the turquoise module, that were potential targets for *M. bovis* to modulate host autophagy. The *CTSS* hub-central gene encodes the proteolytic enzyme cathepsin S, which acts primarily on lysosomes (González-Ruiz et al., 2019). Surprisingly, research has shown that pathogens such as *M. tuberculosis* and *M. bovis* prevent lysosome-autophagosome fusion (autophagosome maturation; Pawar et al., 2016) and lysosome-phagosome fusion (phagosome maturation; Pires et al., 2017) by suppressing *CTSS* gene expression, and prevent autophagy and phagocytosis, respectively. In addition to *VPS33B*, *VPS11* and *VPS18* are key mediators for autophagosome-lysosome fusion, and their dephosphorylation during *M. tuberculosis* infection prevents autophagosome maturation (Rohde et al., 2007; Chandra et al., 2015). Therefore, developing anti-TB therapies based on autophagy targeting can be a key strategy for controlling the intracellular growth and proliferation of pathogenic mycobacteria (Paik et al., 2019).

In conclusion, in the current study, we use a systems biology approach for a deep investigation of the interactions of bAMs and *M. bovis* in order to better understand the molecular regulatory mechanisms underlying bTB and to identify novel insights into immunomodulatory mechanisms inducted by intracellular *M. bovis* for maintaining mycobacterial survival and replication. Combining RNA-seq data and WGCNA module preservation analysis with functional enrichment analysis resulted in the identification of 7 bTB-specific modules in reference samples whose (1) topological properties, such as connectivity patterns and network density, were altered under *M. bovis*-infected conditions, and (2) they were directly biologically related to the bAMs-*M. bovis* interactions such as host immune response, *M. bovis* immune subversion mechanisms, and bTB development. Moreover, the integration of co-expression gene networks based on hub genes of the bTB-specific modules with PPI networks led to the identification of 260 genes that had double centrality in their respective networks (co-expression modules and downstream co-expressed hub genes-based PPI networks). Additionally, our results provided evidence that these hub-central genes played a key role in the fate of *M. bovis* infection and maybe act as the core of several immunosuppressive mechanisms of the *M. bovis*, such as prevention of macrophage phagosome-lysosome fusion, induction of necrosis, inhibition of apoptosis and autophagy, suppression of antigen presentation, modulation of type I IFNs, modulation of IFN-γ production and signaling, modulation of macrophage signaling mechanisms, manipulation of host macrophage metabolism, recruitment of cell surface receptors on the host macrophage, cytosolic escape from the phagosome, and inhibition of ROS production, to escape the host immune response. Notwithstanding this, further research is needed to deep explore the key role of hub-central genes reported in this study to develop novel and more effective therapeutic and diagnostic approaches to control or eradication bTB.

## Data availability statement

The original contributions presented in the study are included in the article/Supplementary material, further inquiries can be directed to the corresponding authors.

## Author contributions

AH and AB conceived the ideas. AH, FS and AB designed the study. AH, AB, HA, and NS analyzed the data. AH, AB, and FS administrated the project. AH, SM, ShM and AB interpreted the data. HA, AH, SaM, ShM, FS and AB validated the data. AH, FS and AB wrote the main manuscript. FR, GJ, and HK helped in writing the manuscript. ShM, HB, MD, AH, and AB reviewed and edited the manuscript. All authors read and approved the final version of manuscript.

## Conflict of interest

The authors declare that the research was conducted in the absence of any commercial or financial relationships that could be construed as a potential conflict of interest.

## Publisher’s note

All claims expressed in this article are solely those of the authors and do not necessarily represent those of their affiliated organizations, or those of the publisher, the editors and the reviewers. Any product that may be evaluated in this article, or claim that may be made by its manufacturer, is not guaranteed or endorsed by the publisher.

## Footnotes

^1^ https://www.bioinformatics.babraham.ac.uk/projects/fastqc/

^2^ https://maayanlab.cloud/Enrichr/

^3^ http://bioinfo.life.hust.edu.cn/AnimalTFDB/#!/

^4^ https://string-db.org/

^5^ https://cytoscape.org/

## Abbreviations

bAMs: Bovine alveolar macrophages
bTB: Bovine tuberculosis
CPM: Count per million
DEGs: Differentially expressed genes
GEO: Gene expression omnibus
GO: Gene ontology
hpi: Hours post infection
IFN: Interferon
KEGG: Kyoto encyclopedia of genes and genomes
MCC: Maximal clique centrality
MM: Module memberships
MTBC: *Mycobacterium tuberculosis* complex
NCBI: National center for biotechnology information
NO: Nitric oxide
PAMPs: Pathogen associated molecular patterns
PPI: Protein–protein interaction
PRRs: Pattern recognition receptors
RNA-seq: RNA sequencing
ROS: Reactive oxygen species
STRING: Search tool for the retrieval of interacting genes
TB: Tuberculosis
TFs: Transcription factors
TOM: Topological overlap matrix
WGCNA: Weighted gene co-expression network analysis

## References

[ref1] AbdallaA. E.EjazH.MahjoobM. O.AlameenA. A. M.AbosalifK. O. A.ElamirM. Y. M.. (2020). Intelligent mechanisms of macrophage apoptosis subversion by mycobacterium. Pathogens 9:218. doi: 10.3390/pathogens9030218, PMID: 32188164PMC7157668

[ref2] AbdelaalH. F. M.ThackerT. C.WadieB.PalmerM. V.TalaatA. M.EhrtS. (2022). Transcriptional profiling of early and late phases of bovine tuberculosis. Infect. Immun. 90:e0031321. doi: 10.1128/iai.00313-21, PMID: 34898250PMC8853682

[ref3] Abo-KadoumM. A.AssadM.AliM. K.UaeM.NzaouS. A. E.GongZ.. (2021). *Mycobacterium tuberculosis* PE17 (Rv1646) promotes host cell apoptosis *via* host chromatin remodeling mediated by reduced H3K9me3 occupancy. Microb. Pathog. 159:105147. doi: 10.1016/j.micpath.2021.105147, PMID: 34400280

[ref4] AiyazM.BipinC.PantulwarV.MugasimangalamR.ShanleyC. A.OrdwayD. J.. (2014). Whole genome response in Guinea pigs infected with the high virulence strain *Mycobacterium tuberculosis* TT372. Tuberculosis 94, 606–615. doi: 10.1016/j.tube.2014.10.001, PMID: 25621360PMC4315170

[ref5] AkiraS.UematsuS.TakeuchiO. (2006). Pathogen recognition and innate immunity. Cells 124, 783–801. doi: 10.1016/j.cell.2006.02.01516497588

[ref6] AlamA.Abubaker BagabirH.SultanA.SiddiquiM. F.ImamN.AlkhananiM. F.. (2022). An integrative network approach to identify common genes for the therapeutics in tuberculosis and its overlapping non-communicable diseases. Front. Pharmacol. 12:770762. doi: 10.3389/fphar.2021.770762, PMID: 35153741PMC8829040

[ref7] AlamA.ImamN.AhmedM. M.TazyeenS.TamkeenN.FarooquiA.. (2019). Identification and classification of differentially expressed genes and network meta-analysis reveals potential molecular signatures associated with tuberculosis. Front. Genet. 10:932. doi: 10.3389/fgene.2019.00932, PMID: 31749827PMC6844239

[ref8] AlamA.ImamN.SiddiquiM. F.AliM. K.AhmedM. M.IshratR. (2021). Human gene expression profiling identifies key therapeutic targets in tuberculosis infection: A systematic network meta-analysis. Infect. Genet. Evol. 87:104649. doi: 10.1016/j.meegid.2020.104649, PMID: 33271338

[ref9] Alcaraz-LópezO. A.Villarreal-MoralesY.Rangel-EscareñoC.Gutiérrez-PabelloJ. A. (2020). Assessment of candidate biomarkers to detect resistance to *Mycobacterium bovis* in Holstein-Friesian cattle. Res. Vet. Sci. 132, 416–425. doi: 10.1016/j.rvsc.2020.07.016, PMID: 32768870

[ref10] AllenS.SotosJ.SylteM. J.CzuprynskiC. J. (2001). Use of hoechst 33342 staining to detect apoptotic changes in bovine mononuclear phagocytes infected with *Mycobacterium avium* subsp. *paratuberculosis*. Clin. Diagn. Lab. Immunol. 8, 460–464. doi: 10.1128/CDLI.8.2.460-464.2001, PMID: 11238240PMC96081

[ref11] AlmE.ArkinA. P. (2003). Biological networks. Curr. Opin. Struct. Biol. 13, 193–202. doi: 10.1016/S0959-440X(03)00031-912727512

[ref12] AlsulaimanyF. A.ZabermawiN. M. O.AlmukadiH.ParambathS. V.ShettyP. J.VaidyanathanV.. (2022). Transcriptome-based molecular networks uncovered interplay between druggable genes of CD8+ T cells and changes in immune cell landscape in patients with pulmonary tuberculosis. Front. Med. 8:812857. doi: 10.3389/fmed.2021.812857, PMID: 35198572PMC8859411

[ref13] AndersS.PylP. T.HuberW. (2014). HTSeq—a python framework to work with high-throughput sequencing data. Bioinformatics 31, 166–169. doi: 10.1093/bioinformatics/btu638, PMID: 25260700PMC4287950

[ref14] AndreuN.PhelanJ.de SessionsP. F.CliffJ. M.ClarkT. G.HibberdM. L. (2017). Primary macrophages and J774 cells respond differently to infection with *Mycobacterium tuberculosis*. Sci. Rep. 7:42225. doi: 10.1038/srep42225, PMID: 28176867PMC5296737

[ref15] Aranday-CortesE.HogarthP. J.KavehD. A.WhelanA. O.Villarreal-RamosB.LalvaniA.. (2012). Transcriptional profiling of disease-induced host responses in bovine tuberculosis and the identification of potential diagnostic biomarkers. PLoS One 7:e30626. doi: 10.1371/journal.pone.0030626, PMID: 22359547PMC3281027

[ref16] ArbuésA.BreesD.ChiboutS.-D.FoxT.KammüllerM.PortevinD. (2020). TNF-α antagonists differentially induce TGF-β1-dependent resuscitation of dormant-like *Mycobacterium tuberculosis*. PLoS Pathog. 16:e1008312. doi: 10.1371/journal.ppat.1008312, PMID: 32069329PMC7048311

[ref17] ArsenaultR. J.MaattanenP.DaigleJ.PotterA.GriebelP.NapperS. (2014). From mouth to macrophage: mechanisms of innate immune subversion by *Mycobacterium avium* subsp. *paratuberculosis*. Vet. Res. 45:54. doi: 10.1186/1297-9716-45-54, PMID: 24885748PMC4046017

[ref18] BachH.PapavinasasundaramK. G.WongD.HmamaZ.Av-GayY. (2008). *Mycobacterium tuberculosis* virulence is mediated by PtpA dephosphorylation of human vacuolar protein sorting 33B. Cell Host Microbe 3, 316–322. doi: 10.1016/j.chom.2008.03.008, PMID: 18474358

[ref19] BaiX.FeldmanN. E.ChmuraK.OvrutskyA. R.SuW.-L.GriffinL.. (2013). Inhibition of nuclear factor-kappa B activation decreases survival of *Mycobacterium tuberculosis* in human macrophages. PLoS One 8:e61925. doi: 10.1371/journal.pone.0061925, PMID: 23634218PMC3636238

[ref20] BaiQ.LiuH.GuoH.LinH.SongX.JinY.. (2020). Identification of hub genes associated with development and microenvironment of hepatocellular carcinoma by weighted gene co-expression network analysis and differential gene expression analysis. Front. Genet. 11:615308. doi: 10.3389/fgene.2020.615308, PMID: 33414813PMC7783465

[ref21] BakhtiarizadehM. R.HosseinpourB.ShahhoseiniM.KorteA.GifaniP. (2018). Weighted gene co-expression network analysis of endometriosis and identification of functional modules associated with its main hallmarks. Front. Genet. 9:453. doi: 10.3389/fgene.2018.00453, PMID: 30369943PMC6194152

[ref22] BakhtiarizadehM. R.MirzaeiS.NorouziM.SheybaniN.Vafaei SadiM. S. (2020). Identification of gene modules and hub genes involved in mastitis development using a systems biology approach. Front. Genet. 11:722. doi: 10.3389/fgene.2020.00722, PMID: 32754201PMC7371005

[ref23] BanksD. A.AhlbrandS. E.HughittV. K.ShahS.Mayer-BarberK. D.VogelS. N.. (2019). *Mycobacterium tuberculosis* inhibits autocrine type I IFN signaling to increase intracellular survival. J. Immunol. 202, 2348–2359. doi: 10.4049/jimmunol.1801303, PMID: 30833347PMC6456408

[ref24] BarabásiA.-L.GulbahceN.LoscalzoJ. (2011). Network medicine: a network-based approach to human disease. Nat. Rev. Genet. 12, 56–68. doi: 10.1038/nrg2918, PMID: 21164525PMC3140052

[ref25] BeckwithK. S.BeckwithM. S.UllmannS.SætraR. S.KimH.MarstadA.. (2020). Plasma membrane damage causes NLRP3 activation and pyroptosis during *Mycobacterium tuberculosis* infection. Nat. Commun. 11:2270. doi: 10.1038/s41467-020-16143-6, PMID: 32385301PMC7210277

[ref26] BeharS. M.MartinC. J.BootyM. G.NishimuraT.ZhaoX.GanH. X.. (2011). Apoptosis is an innate defense function of macrophages against *Mycobacterium tuberculosis*. Mucosal Immunol. 4, 279–287. doi: 10.1038/mi.2011.3, PMID: 21307848PMC3155700

[ref27] BeheraA.JainP.GanguliG.BiswasM.PadhiA.PattanaikK. P.. (2022). *Mycobacterium tuberculosis* acetyltransferase suppresses oxidative stress by inducing peroxisome formation in macrophages. Int. J. Mol. Sci. 23:2584. doi: 10.3390/ijms23052584, PMID: 35269727PMC8909987

[ref28] BellL.PeyperJ. M.GarnettS.TadokeraR.WilkinsonR.MeintjesG.. (2017). TB-IRIS: proteomic analysis of in vitro PBMC responses to *Mycobacterium tuberculosis* and response modulation by dexamethasone. Exp. Mol. Pathol. 102, 237–246. doi: 10.1016/j.yexmp.2017.02.008, PMID: 28209523PMC5446321

[ref29] Benítez-GuzmánA.Arriaga-PizanoL.MoránJ.Gutiérrez-PabelloJ. A. (2018). Endonuclease G takes part in AIF-mediated caspase-independent apoptosis in *Mycobacterium bovis*-infected bovine macrophages. Vet. Res. 49:69. doi: 10.1186/s13567-018-0567-1, PMID: 30021619PMC6052627

[ref30] BenmerzougS.MarinhoF. V.RoseS.MackowiakC.GossetD.SeddaD.. (2018). GM-CSF targeted immunomodulation affects host response to *M. tuberculosis* infection. Sci. Rep. 8:8652. doi: 10.1038/s41598-018-26984-3, PMID: 29872095PMC5988704

[ref31] BiD.NingH.LiuS.QueX.DingK. (2015). Gene expression patterns combined with network analysis identify hub genes associated with bladder cancer. Comput. Biol. Chem. 56, 71–83. doi: 10.1016/j.compbiolchem.2015.04.001, PMID: 25889321

[ref32] BlancoF. C.SoriaM.BiancoM. V.BigiF. (2012). Transcriptional response of peripheral blood mononuclear cells from cattle infected with *Mycobacterium bovis*. PLoS One 7:e41066. doi: 10.1371/journal.pone.0041066, PMID: 22815916PMC3397951

[ref33] BlumenthalA.EhlersS.LauberJ. R.BuerJ.LangeC.GoldmannT.. (2006). The wingless homolog WNT5A and its receptor Frizzled-5 regulate inflammatory responses of human mononuclear cells induced by microbial stimulation. Blood 108, 965–973. doi: 10.1182/blood-2005-12-5046, PMID: 16601243

[ref34] BoechatA. L.OguskuM. M.SadahiroA.dos SantosM. C. (2013). Association between the PTPN22 1858C/T gene polymorphism and tuberculosis resistance. Infect. Genet. Evol. 16, 310–313. doi: 10.1016/j.meegid.2013.02.019, PMID: 23499775

[ref35] BoggiattoP. M.KanipeC. R.PalmerM. V. (2021). Enhanced detection of *Mycobacterium bovis*-specific T cells in experimentally-infected cattle. Front. Vet. Sci. 8:676710. doi: 10.3389/fvets.2021.676710, PMID: 34336973PMC8317970

[ref36] BolgerA. M.LohseM.UsadelB. (2014). Trimmomatic: a flexible trimmer for Illumina sequence data. Bioinformatics 30, 2114–2120. doi: 10.1093/bioinformatics/btu170, PMID: 24695404PMC4103590

[ref37] BorahK.BeyßM.TheorellA.WuH.BasuP.MendumT. A.. (2019). Intracellular *Mycobacterium tuberculosis* exploits multiple host nitrogen sources during growth in human macrophages. Cell Rep. 29, 3580–3591.e4. doi: 10.1016/j.celrep.2019.11.037, PMID: 31825837PMC6915324

[ref38] BrooksM. N.RajaramM. V. S.AzadA. K.AmerA. O.Valdivia-ArenasM. A.ParkJ.-H.. (2011). NOD2 controls the nature of the inflammatory response and subsequent fate of *Mycobacterium tuberculosis* and *M. bovis* BCG in human macrophages. Cell. Microbiol. 13, 402–418. doi: 10.1111/j.1462-5822.2010.01544.x, PMID: 21040358PMC3259431

[ref39] BroschR.GordonS. V.MarmiesseM.BrodinP.BuchrieserC.EiglmeierK.. (2002). A new evolutionary scenario for the *Mycobacterium tuberculosis* complex. Proc. Natl. Acad. Sci. 99, 3684–3689. doi: 10.1073/pnas.052548299, PMID: 11891304PMC122584

[ref40] BuddleB. M.VordermeierH. M.HewinsonR. G.Jr.WR.McShaneH.MizrahiV.. (2016). Experimental infection models of tuberculosis in domestic livestock. Microbiol. Spectrum 4:4.4.66. doi: 10.1128/microbiolspec.TBTB2-0017-201627726786

[ref41] ButlerR. E.BrodinP.JangJ.JangM.-S.RobertsonB. D.GicquelB.. (2012). The balance of apoptotic and necrotic cell death in *Mycobacterium tuberculosis* infected macrophages is not dependent on bacterial virulence. PLoS One 7:e47573. doi: 10.1371/journal.pone.0047573, PMID: 23118880PMC3484146

[ref42] CaiY.YangQ.TangY.ZhangM.LiuH.ZhangG.. (2014). Increased complement C1q level marks active disease in human tuberculosis. PLoS One 9:e92340. doi: 10.1371/journal.pone.0092340, PMID: 24647646PMC3960215

[ref43] CarranzaC.Pedraza-SanchezS.de Oyarzabal-MendezE.TorresM. (2020). Diagnosis for latent tuberculosis infection: new alternatives. Front. Immunol. 11:2006. doi: 10.3389/fimmu.2020.02006, PMID: 33013856PMC7511583

[ref44] CassidyJ. P. (2006). The pathogenesis and pathology of bovine tuberculosis with insights from studies of tuberculosis in humans and laboratory animal models. Vet. Microbiol. 112, 151–161. doi: 10.1016/j.vetmic.2005.11.031, PMID: 16310979

[ref45] CassidyJ. P.BrysonD. G.Gutiérrez CancelaM. M.ForsterF.PollockJ. M.NeillS. D. (2001). Lymphocyte subtypes in experimentally induced early-stage bovine tuberculous lesions. J. Comp. Pathol. 124, 46–51. doi: 10.1053/jcpa.2000.0427, PMID: 11428188

[ref46] CastilloE. F.DekonenkoA.Arko-MensahJ.MandellM. A.DupontN.JiangS.. (2012). Autophagy protects against active tuberculosis by suppressing bacterial burden and inflammation. Proc. Natl. Acad. Sci. 109, E3168–E3176. doi: 10.1073/pnas.1210500109, PMID: 23093667PMC3503152

[ref47] ChaiQ.WangL.LiuC. H.GeB. (2020). New insights into the evasion of host innate immunity by *Mycobacterium tuberculosis*. Cell. Mol. Immunol. 17, 901–913. doi: 10.1038/s41423-020-0502-z, PMID: 32728204PMC7608469

[ref48] ChandraV.BhagyarajE.NanduriR.AhujaN.GuptaP. (2015). NR1D1 ameliorates *Mycobacterium tuberculosis* clearance through regulation of autophagy. Autophagy 11, 1987–1997. doi: 10.1080/15548627.2015.1091140, PMID: 26390081PMC4824569

[ref49] ChandraV.MahajanS.SainiA.DkharH. K.NanduriR.RajE. B.. (2013). Human IL10 gene repression by rev-erbα ameliorates *Mycobacterium tuberculosis* clearance. J. Biol. Chem. 288, 10692–10702. doi: 10.1074/jbc.M113.455915, PMID: 23449984PMC3624449

[ref50] ChandraP.RajmaniR. S.VermaG.BhaveshN. S.KumarD.StallingsC. L. (2016). Targeting drug-sensitive and -resistant strains of *Mycobacterium tuberculosis* by inhibition of SRC family kinases lowers disease burden and pathology. mSphere 1, e00043–e00015. doi: 10.1128/mSphere.00043-15, PMID: 27303736PMC4894694

[ref51] ChatterjeeS.YabajiS. M.RukhlenkoO. S.BhattacharyaB.WaligurskiE.VallavojuN.. (2021). Channeling macrophage polarization by rocaglates increases macrophage resistance to *Mycobacterium tuberculosis*. iScience 24:102845. doi: 10.1016/j.isci.2021.102845, PMID: 34381970PMC8333345

[ref52] ChenZ. (2015). *Mycobacterium tuberculosis* favors its survival by utilizing host ubiquitin to impair innate immunity. Natl. Sci. Rev. 2, 260–261. doi: 10.1093/nsr/nwv034

[ref53] ChenX.CaoX.LeiY.RehemanA.ZhouW.YangB.. (2021a). Distinct persistence fate of *Mycobacterium tuberculosis* in various types of cells. mSystems 6, e00783–e00721. doi: 10.1128/mSystems.00783-2134402643PMC8409741

[ref54] ChenX.KangR.KroemerG.TangD. (2021b). Ferroptosis in infection, inflammation, and immunity. J. Exp. Med. 218:e20210518. doi: 10.1084/jem.20210518, PMID: 33978684PMC8126980

[ref55] ChenJ.LiuC.LiangT.XuG.ZhangZ.LuZ.. (2021). Comprehensive analyses of potential key genes in active tuberculosis: A systematic review. Medicine 100:e26582. doi: 10.1097/md.0000000000026582, PMID: 34397688PMC8322549

[ref56] ChenE. Y.TanC. M.KouY.DuanQ.WangZ.MeirellesG. V.. (2013). Enrichr: interactive and collaborative HTML5 gene list enrichment analysis tool. BMC Bioinf. 14:128. doi: 10.1186/1471-2105-14-128, PMID: 23586463PMC3637064

[ref57] ChenZ.-Y.WangL.GuL.QuR.LowrieD. B.HuZ.. (2020). Decreased expression of CD69 on T cells in tuberculosis infection resisters. Front. Microbiol. 11:1901. doi: 10.3389/fmicb.2020.01901, PMID: 32849474PMC7426741

[ref58] ChenY.WangQ.LinS.LaiJ.LinJ.AoW.. (2021). Meta-analysis of peripheral blood transcriptome datasets reveals a biomarker panel for tuberculosis in patients infected with HIV. Front. Cell. Infect. Microbiol. 11:585919. doi: 10.3389/fcimb.2021.585919, PMID: 33816327PMC8017209

[ref59] ChinC.-H.ChenS.-H.WuH.-H.HoC.-W.KoM.-T.LinC.-Y. (2014). cytoHubba: identifying hub objects and sub-networks from complex interactome. BMC Syst. Biol. 8:S11. doi: 10.1186/1752-0509-8-S4-S11, PMID: 25521941PMC4290687

[ref60] CimminoF.AvitabileM.LasorsaV. A.MontellaA.PezoneL.CantalupoS.. (2019). HIF-1 transcription activity: HIF1A driven response in normoxia and in hypoxia. BMC Med. Genet. 20:37. doi: 10.1186/s12881-019-0767-1, PMID: 30808328PMC6390360

[ref61] ClineM. S.SmootM.CeramiE.KuchinskyA.LandysN.WorkmanC.. (2007). Integration of biological networks and gene expression data using Cytoscape. Nat. Protoc. 2, 2366–2382. doi: 10.1038/nprot.2007.324, PMID: 17947979PMC3685583

[ref62] ColeS. T.BroschR.ParkhillJ.GarnierT.ChurcherC.HarrisD.. (1998). Deciphering the biology of *Mycobacterium tuberculosis* from the complete genome sequence. Nature 393, 537–544. doi: 10.1038/31159, PMID: 9634230

[ref63] CooperA. M.TorradoE. (2012). Protection versus pathology in tuberculosis: recent insights. Curr. Opin. Immunol. 24, 431–437. doi: 10.1016/j.coi.2012.04.008, PMID: 22613092PMC3423558

[ref64] CronanM. R.HughesE. J.BrewerW. J.ViswanathanG.HuntE. G.SinghB.. (2021). A non-canonical type 2 immune response coordinates tuberculous granuloma formation and epithelialization. Cells 184, 1757–1774.e14. doi: 10.1016/j.cell.2021.02.046, PMID: 33761328PMC8055144

[ref65] CummingB. M.RahmanM. A.LamprechtD. A.RohdeK. H.SainiV.AdamsonJ. H.. (2017). *Mycobacterium tuberculosis* arrests host cycle at the G1/S transition to establish long term infection. PLoS Pathog. 13:e1006389. doi: 10.1371/journal.ppat.1006389, PMID: 28542477PMC5456404

[ref66] DasS.MeherP. K.RaiA.BharL. M.MandalB. N. (2017). Statistical approaches for gene selection, hub gene identification and module interaction in gene co-expression network analysis: an application to aluminum stress in soybean (Glycine max L.). PLoS One 12:e0169605. doi: 10.1371/journal.pone.0169605, PMID: 28056073PMC5215982

[ref67] DayC. L.AbrahamsD. A.LerumoL.Janse van RensburgE.StoneL.O’rieT.. (2011). Functional capacity of *Mycobacterium tuberculosis*-specific T cell responses in humans is associated with mycobacterial load. J. Immunol. 187, 2222–2232. doi: 10.4049/jimmunol.1101122, PMID: 21775682PMC3159795

[ref68] DenisM.KeenD. L.ParlaneN. A.StorsetA. K.BuddleB. M. (2007). Bovine natural killer cells restrict the replication of *Mycobacterium bovis* in bovine macrophages and enhance IL-12 release by infected macrophages. Tuberculosis 87, 53–62. doi: 10.1016/j.tube.2006.03.005, PMID: 16730232

[ref69] DenisM.WedlockD. N.BuddleB. M. (2005). IFN-γ enhances bovine macrophage responsiveness to *Mycobacterium bovis*: impact on bacterial replication, cytokine release and macrophage apoptosis. Immunol. Cell Biol. 83, 643–650. doi: 10.1111/j.1440-1711.2005.01386.x, PMID: 16266317

[ref70] DivangahiM.MostowyS.CoulombeF.KozakR.GuillotL.VeyrierF.. (2008). NOD2-deficient mice have impaired resistance to *Mycobacterium tuberculosis* infection through defective innate and adaptive immunity. J. Immunol. 181, 7157–7165. doi: 10.4049/jimmunol.181.10.7157, PMID: 18981137

[ref71] DjelouadjiZ.RaoultD.DrancourtM. (2011). Palaeogenomics of *Mycobacterium tuberculosis*: epidemic bursts with a degrading genome. Lancet Infect. Dis. 11, 641–650. doi: 10.1016/S1473-3099(11)70093-7, PMID: 21672667

[ref72] DongW.WangG.FengJ.LiP.WangR.LuH.. (2022). MiR-25 blunts autophagy and promotes the survival of *Mycobacterium tuberculosis* by regulating NPC1. iScience 25:104279. doi: 10.1016/j.isci.2022.104279, PMID: 35586071PMC9108763

[ref73] DuanP.BonewaldL. F. (2016). The role of the wnt/β-catenin signaling pathway in formation and maintenance of bone and teeth. Int. J. Biochem. Cell Biol. 77, 23–29. doi: 10.1016/j.biocel.2016.05.015, PMID: 27210503PMC4958569

[ref74] DuttaN. K.MehraS.MartinezA. N.AlvarezX.RennerN. A.MoriciL. A.. (2012). The stress-response factor SigH modulates the interaction between *Mycobacterium tuberculosis* and host phagocytes. PLoS One 7:e28958. doi: 10.1371/journal.pone.0028958, PMID: 22235255PMC3250399

[ref75] EhlersS. (2003). Role of tumour necrosis factor (TNF) in host defence against tuberculosis: implications for immunotherapies targeting TNF. Ann. Rheum. Dis. 62:37ii. doi: 10.1136/ard.62.suppl_2.ii37, PMID: 14532147PMC1766754

[ref76] EissingT.KuepferL.BeckerC.BlockM.CoboekenK.GaubT.. (2011). A computational systems biology software platform for multiscale modeling and simulation: integrating whole-body physiology, disease biology, and molecular reaction networks. Front. Physiol. 2:4. doi: 10.3389/fphys.2011.00004, PMID: 21483730PMC3070480

[ref77] ElkingtonP.ShiomiT.BreenR.NuttallR. K.Ugarte-GilC. A.WalkerN. F.. (2011). MMP-1 drives immunopathology in human tuberculosis and transgenic mice. J. Clin. Invest. 121, 1827–1833. doi: 10.1172/JCI45666, PMID: 21519144PMC3083790

[ref78] Esquivel-SolísH.Quiñones-FalconiF.Zarain-HerzbergA.Amieva-FernándezR. I.López-VidalY. (2009). Impaired activation of Stat1 and c-Jun as a possible defect in macrophages of patients with active tuberculosis. Clin. Exp. Immunol. 158, 45–54. doi: 10.1111/j.1365-2249.2009.03985.x, PMID: 19737230PMC2759058

[ref79] FangL.LinW.JiaH.GaoX.SuiX.GuoX.. (2020). Potential diagnostic value of the peripheral blood mononuclear cell transcriptome from cattle with bovine tuberculosis. Front. Vet. Sci. 7:295. doi: 10.3389/fvets.2020.00295, PMID: 32528988PMC7266948

[ref80] FayyaziA.EichmeyerB.SoruriA.SchweyerS.HermsJ.SchwarzP.. (2000). Apoptosis of macrophages and T cells in tuberculosis associated caseous necrosis. J. Pathol. 191, 417–425. doi: 10.1002/1096-9896(2000)9999:9999<::AID-PATH664>3.0.CO;2-R, PMID: 10918217

[ref81] FlynnJ. L.ChanJ.TrieboldK. J.DaltonD. K.StewartT. A.BloomB. R. (1993). An essential role for interferon gamma in resistance to *Mycobacterium tuberculosis* infection. J. Exp. Med. 178, 2249–2254. doi: 10.1084/jem.178.6.2249, PMID: 7504064PMC2191274

[ref82] FrancoL. H.NairV. R.ScharnC. R.XavierR. J.TorrealbaJ. R.ShilohM. U.. (2017). The ubiquitin ligase smurf1 functions in selective autophagy of *Mycobacterium tuberculosis* and anti-tuberculous host defense. Cell Host Microbe 21, 59–72. doi: 10.1016/j.chom.2016.11.002, PMID: 28017659PMC5699477

[ref83] FrancoE. F.RanaP.Queiroz CavalcanteA. L.da SilvaA. L.Gomide AC. P.Carneiro FoladorA. R.. (2020). Co-expression networks for causal gene identification based on RNA-seq data of Corynebacterium pseudotuberculosis. Genes 11:794. doi: 10.3390/genes11070794, PMID: 32674507PMC7397307

[ref84] GallegosA. M.van HeijstJ. W. J.SamsteinM.SuX.PamerE. G.GlickmanM. S. (2011). A gamma interferon independent mechanism of CD4 T cell mediated control of *M. tuberculosis* infection in vivo. PLoS Pathog. 7:e1002052. doi: 10.1371/journal.ppat.1002052, PMID: 21625591PMC3098235

[ref85] GarnierT.EiglmeierK.CamusJ.-C.MedinaN.MansoorH.PryorM.. (2003). The complete genome sequence of *Mycobacterium bovis*. Proc. Natl. Acad. Sci. 100, 7877–7882. doi: 10.1073/pnas.1130426100, PMID: 12788972PMC164681

[ref86] GautamU. S.ForemanT. W.BucsanA. N.VeatchA. V.AlvarezX.AdekambiT.. (2018). In vivo inhibition of tryptophan catabolism reorganizes the tuberculoma and augments immune-mediated control of *Mycobacterium tuberculosis*. Proc. Natl. Acad. Sci. 115, E62–E71. doi: 10.1073/pnas.1711373114, PMID: 29255022PMC5776797

[ref87] GautamU. S.MehraS.AhsanM. H.AlvarezX.NiuT.KaushalD. (2014). Role of TNF in the altered interaction of dormant *Mycobacterium tuberculosis* with host macrophages. PLoS One 9:e95220. doi: 10.1371/journal.pone.0095220, PMID: 24743303PMC3990579

[ref88] GebremicaelG.KassaD.AlemayehuY.GebreegziaxierA.KassahunY.van BaarleD.. (2019). Gene expression profiles classifying clinical stages of tuberculosis and monitoring treatment responses in Ethiopian HIV-negative and HIV-positive cohorts. PLoS One 14:e0226137. doi: 10.1371/journal.pone.0226137, PMID: 31821366PMC6903757

[ref89] GebremicaelG.KassaD.QuintenE.AlemayehuY.GebreegziaxierA.BelayY.. (2018). Host gene expression kinetics during treatment of tuberculosis in HIV-coinfected individuals is independent of highly active antiretroviral therapy. J. Infect. Dis. 218, 1833–1846. doi: 10.1093/infdis/jiy404, PMID: 29982697

[ref90] GehringA. J.RojasR. E.CanadayD. H.LakeyD. L.HardingC. V.BoomW. H. (2003). The *Mycobacterium tuberculosis* 19-kilodalton lipoprotein inhibits gamma interferon-regulated HLA-DR and FcγR1 on human macrophages through toll-like receptor 2. Infect. Immun. 71, 4487–4497. doi: 10.1128/IAI.71.8.4487-4497.2003, PMID: 12874328PMC166015

[ref91] GeroldG.ZychlinskyA.de DiegoJ. L. (2007). What is the role of toll-like receptors in bacterial infections? Semin. Immunol. 19, 41–47. doi: 10.1016/j.smim.2006.12.00317280841

[ref92] GongW.-P.LiangY.LingY.-B.ZhangJ.-X.YangY.-R.WangL.. (2020). Effects of mycobacterium vaccae vaccine in a mouse model of tuberculosis: protective action and differentially expressed genes. Mil. Med. Res. 7:25. doi: 10.1186/s40779-020-00258-4, PMID: 32493477PMC7268289

[ref93] González-RuizS.StrillacciM. G.Durán-AguilarM.Cantó-AlarcónG. J.Herrera-RodríguezS. E.BagnatoA.. (2019). Genome-wide association study in mexican Holstein cattle reveals novel quantitative trait loci regions and confirms mapped loci for resistance to bovine tuberculosis. Animals 9:636. doi: 10.3390/ani9090636, PMID: 31480266PMC6769677

[ref94] GouzyA.PoquetY.NeyrollesO. (2014). Amino acid capture and utilization within the *Mycobacterium tuberculosis* phagosome. Future Microbiol. 9, 631–637. doi: 10.2217/fmb.14.28, PMID: 24957090

[ref95] GreenJ. A.ElkingtonP. T.PenningtonC. J.RoncaroliF.DholakiaS.MooresR. C.. (2010). *Mycobacterium tuberculosis* upregulates microglial matrix metalloproteinase-1 and -3 expression and secretion *via* NF-κB– and activator protein-1–dependent monocyte networks. J. Immunol. 184, 6492–6503. doi: 10.4049/jimmunol.0903811, PMID: 20483790

[ref97] Gutiérrez-PabelloJ. A.McMurrayD. N.AdamsL. G. (2002). Upregulation of thymosin β-10 by *Mycobacterium bovis* infection of bovine macrophages is associated with apoptosis. Infect. Immun. 70, 2121–2127. doi: 10.1128/IAI.70.4.2121-2127.2002, PMID: 11895978PMC127845

[ref98] HaS.-H.ChoiH.ParkJ.-Y.AbekuraF.LeeY.-C.KimJ.-R.. (2020). *Mycobacterium tuberculosis*–secreted protein, ESAT-6, inhibits lipopolysaccharide-induced MMP-9 expression and inflammation through NF-κB and MAPK signaling in raw 264.7 macrophage cells. Inflammation 43, 54–65. doi: 10.1007/s10753-019-01087-x, PMID: 31720987

[ref99] HallT. J.MullenM. P.McHugoG. P.KillickK. E.RingS. C.BerryD. P.. (2021). Integrative genomics of the mammalian alveolar macrophage response to intracellular mycobacteria. BMC Genomics 22:343. doi: 10.1186/s12864-021-07643-w, PMID: 33980141PMC8117616

[ref100] HallT. J.VernimmenD.BrowneJ. A.MullenM. P.GordonS. V.MacHughD. E.. (2020). Alveolar macrophage chromatin is modified to orchestrate host response to *Mycobacterium bovis* infection. Front. Genet. 10:1386. doi: 10.3389/fgene.2019.01386, PMID: 32117424PMC7020904

[ref101] HanH. (2019). Identification of several key genes by microarray data analysis of bovine mammary gland epithelial cells challenged with Escherichia coli and Staphylococcus aureus. Gene 683, 123–132. doi: 10.1016/j.gene.2018.10.004, PMID: 30291872

[ref102] HarperJ.SkerryC.DavisS. L.TasneenR.WeirM.KramnikI.. (2011). Mouse model of necrotic tuberculosis granulomas develops hypoxic lesions. J. Infect. Dis. 205, 595–602. doi: 10.1093/infdis/jir786, PMID: 22198962PMC3266133

[ref103] HasankhaniA.BahramiA.SheybaniN.AriaB.HematiB.FatehiF.. (2021a). Differential co-expression network analysis reveals key hub-high traffic genes as potential therapeutic targets for COVID-19 pandemic. Front. Immunol. 12:789317. doi: 10.3389/fimmu.2021.789317, PMID: 34975885PMC8714803

[ref104] HasankhaniA.BahramiA.SheybaniN.FatehiF.AbadehR.Ghaem Maghami FarahaniH.. (2021b). Integrated network analysis to identify key modules and potential hub genes involved in bovine respiratory disease: A systems biology approach. Front. Genet. 12:753839. doi: 10.3389/fgene.2021.753839, PMID: 34733317PMC8559434

[ref105] HeidariM.PakdelA.BakhtiarizadehM. R.DehghanianF. (2021). Integrated analysis of lncRNAs, mRNAs, and TFs to identify regulatory networks underlying MAP infection in cattle. Front. Genet. 12:668448. doi: 10.3389/fgene.2021.668448, PMID: 34290737PMC8287970

[ref106] HoodL.HeathJ. R.PhelpsM. E.LinB. (2004). Systems biology and new technologies enable predictive and preventative medicine. Science 306, 640–643. doi: 10.1126/science.1104635, PMID: 15499008

[ref107] HuH.MiaoY.-R.JiaL.-H.YuQ.-Y.ZhangQ.GuoA.-Y. (2018). AnimalTFDB 3.0: a comprehensive resource for annotation and prediction of animal transcription factors. Nucleic Acids Res. 47, D33–D38. doi: 10.1093/nar/gky822, PMID: 30204897PMC6323978

[ref108] HuangD.BaoL. (2016). *Mycobacterium tuberculosis* EspB protein suppresses interferon-γ-induced autophagy in murine macrophages. J. Microbiol. Immunol. Infect. 49, 859–865. doi: 10.1016/j.jmii.2014.11.008, PMID: 25641595

[ref109] HuangL.YeK.McGeeM. C.NidetzN. F.ElmoreJ. P.LimperC. B.. (2020). Interleukin-2-inducible T-cell kinase deficiency impairs early pulmonary protection against *Mycobacterium tuberculosis* infection. Front. Immunol. 10:3103. doi: 10.3389/fimmu.2019.03103, PMID: 32038633PMC6993117

[ref110] HussainT.ZhaoD.ShahS. Z. A.SabirN.WangJ.LiaoY.. (2019a). Nilotinib: A tyrosine kinase inhibitor mediates resistance to intracellular mycobacterium *via* regulating autophagy. Cells 8:506. doi: 10.3390/cells8050506, PMID: 31130711PMC6562972

[ref111] HussainT.ZhaoD.ShahS. Z. A.SabirN.WangJ.LiaoY.. (2019b). PP2Ac modulates AMPK-mediated induction of autophagy in *Mycobacterium bovis*-infected macrophages. Int. J. Mol. Sci. 20:6030. doi: 10.3390/ijms20236030, PMID: 31795474PMC6928646

[ref112] IizasaE. I.ChumaY.UematsuT.KubotaM.KawaguchiH.UmemuraM.. (2021). TREM2 is a receptor for non-glycosylated mycolic acids of mycobacteria that limits anti-mycobacterial macrophage activation. Nat. Commun. 12:2299. doi: 10.1038/s41467-021-22620-3, PMID: 33863908PMC8052348

[ref113] ImaiK.Kurita-OchiaiT.OchiaiK. (2003). *Mycobacterium bovis* bacillus Calmette-Gueérin infection promotes SOCS induction and inhibits IFN-γ-stimulated JAK/STAT signaling in J774 macrophages. FEMS Immunol. Med. Microbiol. 39, 173–180. doi: 10.1016/s0928-8244(03)00231-1, PMID: 14625101

[ref114] Jaime-LaraR. B.RoyA.WangY.StanfillA.CashionA. K.JosephP. V. (2020). Gene co-expression networks are associated with obesity-related traits in kidney transplant recipients. BMC Med. Genet. 13:37. doi: 10.1186/s12920-020-0702-5, PMID: 32151267PMC7063809

[ref115] JayaswalS.KamalM. A.DuaR.GuptaS.MajumdarT.DasG.. (2010). Identification of host-dependent survival factors for intracellular *Mycobacterium tuberculosis* through an siRNA screen. PLoS Pathog. 6:e1000839. doi: 10.1371/journal.ppat.1000839, PMID: 20419122PMC2855445

[ref116] JensenK.GallagherI. J.JohnstonN.WelshM.SkuceR.WilliamsJ. L.. (2018). Variation in the early host-pathogen interaction of bovine macrophages with divergent *Mycobacterium bovis* strains in the United Kingdom. Infect. Immun. 86, e00385–e00317. doi: 10.1128/IAI.00385-17, PMID: 29263113PMC5820943

[ref117] JensenK.StevensJ. M.GlassE. J. (2019). Interleukin 10 knock-down in bovine monocyte-derived macrophages has distinct effects during infection with two divergent strains of *Mycobacterium bovis*. PLoS One 14:e0222437. doi: 10.1371/journal.pone.0222437, PMID: 31527895PMC6748433

[ref118] JenumS.BakkenR.DhanasekaranS.MukherjeeA.LodhaR.SinghS.. (2016). BLR1 and FCGR1A transcripts in peripheral blood associate with the extent of intrathoracic tuberculosis in children and predict treatment outcome. Sci. Rep. 6:38841. doi: 10.1038/srep38841, PMID: 27941850PMC5150239

[ref119] JiangD.WubuliA.HuX.IkramullahS.MaimaitiA.ZhangW.. (2015). The variations of IL-23R are associated with susceptibility and severe clinical forms of pulmonary tuberculosis in Chinese Uygurs. BMC Infect. Dis. 15:550. doi: 10.1186/s12879-015-1284-2, PMID: 26626589PMC4665827

[ref120] JonesG. J.PirsonC.HewinsonR. G.VordermeierH. M. (2010). Simultaneous measurement of antigen-stimulated interleukin-1β and gamma interferon production enhances test sensitivity for the detection of *Mycobacterium bovis* infection in cattle. Clin. Vaccine Immunol. 17, 1946–1951. doi: 10.1128/CVI.00377-10, PMID: 20926697PMC3008179

[ref121] JoshiA.RienksM.TheofilatosK.MayrM. (2021). Systems biology in cardiovascular disease: a multiomics approach. Nat. Rev. Cardiol. 18, 313–330. doi: 10.1038/s41569-020-00477-1, PMID: 33340009

[ref122] JuárezE.CarranzaC.Hernández-SánchezF.León-ContrerasJ. C.Hernández-PandoR.EscobedoD.. (2012). NOD2 enhances the innate response of alveolar macrophages to *Mycobacterium tuberculosis* in humans. Eur. J. Immunol. 42, 880–889. doi: 10.1002/eji.201142105, PMID: 22531915

[ref123] KahnM. (2014). Can we safely target the WNT pathway? Nat. Rev. Drug Discov. 13, 513–532. doi: 10.1038/nrd4233, PMID: 24981364PMC4426976

[ref124] KangD. D.LinY.MorenoJ.-R.RandallT. D.KhaderS. A. (2011). Profiling early lung immune responses in the mouse model of tuberculosis. PLoS One 6:e16161. doi: 10.1371/journal.pone.0016161, PMID: 21249199PMC3020951

[ref125] KanipeC.PalmerM. V. (2020). *Mycobacterium bovis* and you: A comprehensive look at the bacteria, its similarities to *Mycobacterium tuberculosis*, and its relationship with human disease. Tuberculosis 125:102006. doi: 10.1016/j.tube.2020.102006, PMID: 33032093

[ref126] KatiyarA.SinghH.AzadK. K. (2018). Identification of missing carbon fixation enzymes as potential drug targets in *Mycobacterium tuberculosis*. J. Integr. Bioinf. 15:20170041. doi: 10.1515/jib-2017-0041, PMID: 30218604PMC6340126

[ref127] KaufmannS. H. E.LiébanaE.GirvinR. M.WelshM.NeillS. D.PollockJ. M. (1999). Generation of CD8+ T-cell responses to *Mycobacterium bovis* and mycobacterial antigen in experimental bovine tuberculosis. Infect. Immun. 67, 1034–1044. doi: 10.1128/IAI.67.3.1034-1044.1999, PMID: 10024540PMC96426

[ref128] KeaneJ.Balcewicz-SablinskaM. K.RemoldH. G.ChuppG. L.MeekB. B.FentonM. J.. (1997). Infection by *Mycobacterium tuberculosis* promotes human alveolar macrophage apoptosis. Infect. Immun. 65, 298–304. doi: 10.1128/iai.65.1.298-304.1997, PMID: 8975927PMC174591

[ref129] KeaneJ.RemoldH. G.KornfeldH. (2000). Virulent *Mycobacterium tuberculosis* strains evade apoptosis of infected alveolar macrophages. J. Immunol. 164, 2016–2020. doi: 10.4049/jimmunol.164.4.2016, PMID: 10657653

[ref130] KennedyH. E.WelshM. D.BrysonD. G.CassidyJ. P.ForsterF. I.HowardC. J.. (2002). Modulation of immune responses to *Mycobacterium bovis* in cattle depleted of WC1+ γδ T cells. Infect. Immun. 70, 1488–1500. doi: 10.1128/IAI.70.3.1488-1500.2002, PMID: 11854237PMC127737

[ref131] KhanN.DowneyJ.SanzJ.KaufmannE.BlankenhausB.PacisA.. (2020). *M. Tuberculosis* reprograms hematopoietic stem cells to limit myelopoiesis and impair trained immunity. Cells 183, 752–770.e22. doi: 10.1016/j.cell.2020.09.062, PMID: 33125891PMC7599081

[ref132] KhanN.PahariS.VidyarthiA.AqdasM.AgrewalaJ. N. (2016). Stimulation through CD40 and TLR-4 is an effective host directed therapy against *Mycobacterium tuberculosis*. Front. Immunol. 7:386. doi: 10.3389/fimmu.2016.00386, PMID: 27729911PMC5037235

[ref133] KillickK. E.BrowneJ. A.ParkS. D. E.MageeD. A.MartinI.MeadeK. G.. (2011). Genome-wide transcriptional profiling of peripheral blood leukocytes from cattle infected with *Mycobacterium bovis* reveals suppression of host immune genes. BMC Genomics 12:611. doi: 10.1186/1471-2164-12-611, PMID: 22182502PMC3292584

[ref134] KillickK. E.MageeD. A.ParkS. D. E.TaraktsoglouM.BrowneJ. A.ConlonK. M.. (2014). Key hub and bottleneck genes differentiate the macrophage response to virulent and attenuated *Mycobacterium bovis*. Front. Immunol. 5:422. doi: 10.3389/fimmu.2014.00422, PMID: 25324841PMC4181336

[ref135] KillickK. E.Ní CheallaighC.O'FarrellyC.HokampK.MacHughD. E.HarrisJ. (2013). Receptor-mediated recognition of mycobacterial pathogens. Cell. Microbiol. 15, 1484–1495. doi: 10.1111/cmi.12161, PMID: 23795683

[ref136] KimD.PaggiJ. M.ParkC.BennettC.SalzbergS. L. (2019). Graph-based genome alignment and genotyping with HISAT2 and HISAT-genotype. Nat. Biotechnol. 37, 907–915. doi: 10.1038/s41587-019-0201-4, PMID: 31375807PMC7605509

[ref137] KimmeyJ. M.CampbellJ. A.WeissL. A.MonteK. J.LenschowD. J.StallingsC. L. (2017). The impact of ISGylation during *Mycobacterium tuberculosis* infection in mice. Microbes Infect. 19, 249–258. doi: 10.1016/j.micinf.2016.12.006, PMID: 28087453PMC5403610

[ref138] KleppL. I.EirinM. E.GarbaccioS.SoriaM.BigiF.BlancoF. C. (2019). Identification of bovine tuberculosis biomarkers to detect tuberculin skin test and IFNγ release assay false negative cattle. Res. Vet. Sci. 122, 7–14. doi: 10.1016/j.rvsc.2018.10.016, PMID: 30447501

[ref139] KongY.FengZ.-C.ZhangY.-L.LiuX.-F.MaY.ZhaoZ.-M.. (2020). Identification of immune-related genes contributing to the development of glioblastoma using weighted gene co-expression network analysis. Front. Immunol. 11:1281. doi: 10.3389/fimmu.2020.01281, PMID: 32765489PMC7378359

[ref140] KönigshoffM.EickelbergO. (2010). WNT signaling in lung disease. Am. J. Respir. Cell Mol. Biol. 42, 21–31. doi: 10.1165/rcmb.2008-0485TR19329555

[ref141] KooM.-S.SubbianS.KaplanG. (2012). Strain specific transcriptional response in *Mycobacterium tuberculosis* infected macrophages. Cell Commun. Signaling 10:2. doi: 10.1186/1478-811X-10-2, PMID: 22280836PMC3317440

[ref142] KrutzikS. R.ModlinR. L. (2004). The role of toll-like receptors in combating mycobacteria. Semin. Immunol. 16, 35–41. doi: 10.1016/j.smim.2003.10.005, PMID: 14751762

[ref143] KumarM.SahuS. K.KumarR.SubuddhiA.MajiR. K.JanaK.. (2015). MicroRNA let-7 modulates the immune response to *Mycobacterium tuberculosis* infection *via* control of A20, an inhibitor of the NF-κB pathway. Cell Host Microbe 17, 345–356. doi: 10.1016/j.chom.2015.01.007, PMID: 25683052

[ref144] LandesM. B.RajaramM. V. S.NguyenH.SchlesingerL. S. (2015). Role for NOD2 in *Mycobacterium tuberculosis*-induced iNOS expression and NO production in human macrophages. J. Leukoc. Biol. 97, 1111–1119. doi: 10.1189/jlb.3A1114-557R, PMID: 25801769PMC4438743

[ref145] LangfelderP.HorvathS. (2008). WGCNA: an R package for weighted correlation network analysis. BMC Bioinf. 9:559. doi: 10.1186/1471-2105-9-559, PMID: 19114008PMC2631488

[ref146] LangfelderP.LuoR.OldhamM. C.HorvathS. (2011). Is my network module preserved and reproducible? PLoS Comput. Biol. 7:e1001057. doi: 10.1371/journal.pcbi.1001057, PMID: 21283776PMC3024255

[ref147] LavalettL.RodriguezH.OrtegaH.SadeeW.SchlesingerL. S.BarreraL. F. (2017). Alveolar macrophages from tuberculosis patients display an altered inflammatory gene expression profile. Tuberculosis 107, 156–167. doi: 10.1016/j.tube.2017.08.012, PMID: 29050765

[ref148] LawC. W.ChenY.ShiW.SmythG. K. (2014). Voom: precision weights unlock linear model analysis tools for RNA-seq read counts. Genome Biol. 15:R29. doi: 10.1186/gb-2014-15-2-r29, PMID: 24485249PMC4053721

[ref149] LechartierB.RybnikerJ.ZumlaA.ColeS. T. (2014). Tuberculosis drug discovery in the post-post-genomic era. EMBO Mol. Med. 6, 158–168. doi: 10.1002/emmm.201201772, PMID: 24401837PMC3927952

[ref150] LeeW.VanderVenB. C.FaheyR. J.RussellD. G. (2013). Intracellular *Mycobacterium tuberculosis* exploits host-derived fatty acids to limit metabolic stress. J. Biol. Chem. 288, 6788–6800. doi: 10.1074/jbc.M112.445056, PMID: 23306194PMC3591590

[ref151] LiL.-L.DaiB.SunY.-H.ZhangT.-T. (2020). The activation of IL-17 signaling pathway promotes pyroptosis in pneumonia-induced sepsis. Ann. Transl. Med. 8:674. doi: 10.21037/atm-19-1739, PMID: 32617294PMC7327349

[ref152] LiM.GaoH.WangJ.WuF.-X. (2018). Control principles for complex biological networks. Brief. Bioinform. 20, 2253–2266. doi: 10.1093/bib/bby08830239577

[ref153] LiS.LiuX.LiuT.MengX.YinX.FangC.. (2017). Identification of biomarkers correlated with the TNM staging and overall survival of patients with bladder cancer. Front. Physiol. 8:947. doi: 10.3389/fphys.2017.00947, PMID: 29234286PMC5712410

[ref154] LiF.LuoJ.XuH.WangY.JiangW.ChangK.. (2020). Early secreted antigenic target 6-kDa from *Mycobacterium tuberculosis* enhanced the protective innate immunity of macrophages partially *via* HIF1α. Biochem. Biophys. Res. Commun. 522, 26–32. doi: 10.1016/j.bbrc.2019.11.045, PMID: 31735338

[ref155] LiL.LvJ.HeY.WangZ. (2020). Gene network in pulmonary tuberculosis based on bioinformatic analysis. BMC Infect. Dis. 20:612. doi: 10.1186/s12879-020-05335-6, PMID: 32811479PMC7436983

[ref156] LiL.QiaoD.FuX.LaoS.ZhangX.WuC. (2011). Identification of M.tuberculosis-specific Th1 cells expressing CD69 generated in vivo in pleural fluid cells from patients with tuberculous pleurisy. PLoS One 6:e23700. doi: 10.1371/journal.pone.0023700, PMID: 21887301PMC3161751

[ref157] LiP.WangR.DongW.HuL.ZongB.ZhangY.. (2017). Comparative proteomics analysis of human macrophages infected with virulent *Mycobacterium bovis*. Front. Cell. Infect. Microbiol. 7:65. doi: 10.3389/fcimb.2017.00065, PMID: 28337427PMC5343028

[ref158] LiH.WeiS.FangY.LiM.LiX.LiZ.. (2017). Quantitative proteomic analysis of host responses triggered by *Mycobacterium tuberculosis* infection in human macrophage cells. Acta Biochim. Biophys. Sin. 49, 835–844. doi: 10.1093/abbs/gmx080, PMID: 28910983

[ref159] LiC.XuJ. (2019). Feature selection with the fisher score followed by the maximal clique centrality algorithm can accurately identify the hub genes of hepatocellular carcinoma. Sci. Rep. 9:17283. doi: 10.1038/s41598-019-53471-0, PMID: 31754223PMC6872594

[ref160] LiJ.ZhouD.QiuW.ShiY.YangJ.-J.ChenS.. (2018). Application of weighted gene co-expression network analysis for data from paired design. Sci. Rep. 8:622. doi: 10.1038/s41598-017-18705-z, PMID: 29330528PMC5766625

[ref161] LiangT.ChenJ.XuG.ZhangZ.XueJ.ZengH.. (2022). Ferroptosis-related gene SOCS1, a marker for tuberculosis diagnosis and treatment, involves in macrophage polarization and facilitates bone destruction in tuberculosis. Tuberculosis 132:102140. doi: 10.1016/j.tube.2021.102140, PMID: 34856472

[ref162] LinY.ZhangY.YuH.TianR.WangG.LiF. (2019). Identification of unique key genes and miRNAs in latent tuberculosis infection by network analysis. Mol. Immunol. 112, 103–114. doi: 10.1016/j.molimm.2019.04.032, PMID: 31082644

[ref163] LinJ.ZhaoD.WangJ.WangY.LiH.YinX.. (2015). Transcriptome changes upon in vitro challenge with *Mycobacterium bovis* in monocyte-derived macrophages from bovine tuberculosis-infected and healthy cows. Vet. Immunol. Immunopathol. 163, 146–156. doi: 10.1016/j.vetimm.2014.12.001, PMID: 25550244

[ref164] LiuY.LiJ.-Y.ChenS.-T.HuangH.-R.CaiH. (2016). The rLrp of *Mycobacterium tuberculosis* inhibits proinflammatory cytokine production and downregulates APC function in mouse macrophages *via* a TLR2-mediated PI3K/Akt pathway activation-dependent mechanism. Cell. Mol. Immunol. 13, 729–745. doi: 10.1038/cmi.2015.58, PMID: 26166760PMC5101441

[ref165] LooY.-M.GaleM.Jr. (2011). Immune signaling by RIG-I-like receptors. Immunity 34, 680–692. doi: 10.1016/j.immuni.2011.05.003, PMID: 21616437PMC3177755

[ref166] LooneyM.LorencR.HalushkaM. K.KarakousisP. C. (2021). Key macrophage responses to infection with *Mycobacterium tuberculosis* are co-regulated by microRNAs and DNA methylation. Front. Immunol. 12:685237. doi: 10.3389/fimmu.2021.685237, PMID: 34140955PMC8204050

[ref167] LuL.WeiR.BhaktaS.WaddellS. J.BoixE. (2021). Weighted gene co-expression network analysis identifies key modules and hub genes associated with mycobacterial infection of human macrophages. Antibiotics 10:97. doi: 10.3390/antibiotics10020097, PMID: 33498280PMC7909288

[ref168] LuC.WuJ.WangH.WangS.DiaoN.WangF.. (2011). Novel biomarkers distinguishing active tuberculosis from latent infection identified by gene expression profile of peripheral blood mononuclear cells. PLoS One 6:e24290. doi: 10.1371/journal.pone.0024290, PMID: 21904626PMC3164189

[ref169] LuQ.ZhangW.FangJ.ZhengJ.DongC.XiongS. (2020). *Mycobacterium tuberculosis* Rv1096, facilitates mycobacterial survival by modulating the NF-κB/MAPK pathway as peptidoglycan N-deacetylase. Mol. Immunol. 127, 47–55. doi: 10.1016/j.molimm.2020.08.005, PMID: 32927163

[ref170] LubbersR.SutherlandJ. S.GolettiD.de PausR. A.van MoorselC. H. M.VeltkampM.. (2018). Complement component C1q as serum biomarker to detect active tuberculosis. Front. Immunol. 9:2427. doi: 10.3389/fimmu.2018.02427, PMID: 30405622PMC6206241

[ref171] MaJ.GuiH.TangY.DingY.QianG.YangM.. (2021). In silico identification of 10 hub genes and an miRNA–mRNA regulatory network in acute Kawasaki disease. Front. Genet. 12:585058. doi: 10.3389/fgene.2021.585058, PMID: 33868359PMC8044791

[ref172] MaY.HanF.LiangJ.YangJ.ShiJ.XueJ.. (2016). A species-specific activation of toll-like receptor signaling in bovine and sheep bronchial epithelial cells triggered by mycobacterial infections. Mol. Immunol. 71, 23–33. doi: 10.1016/j.molimm.2016.01.004, PMID: 26802731

[ref173] MacHughD. E.GormleyE.ParkS. D. E.BrowneJ. A.TaraktsoglouM.O’FarrellyC.. (2009). Gene expression profiling of the host response to *Mycobacterium bovis* infection in cattle. Transbound. Emerg. Dis. 56, 204–214. doi: 10.1111/j.1865-1682.2009.01082.x, PMID: 19486308

[ref174] MacHughD. E.TaraktsoglouM.KillickK. E.NalpasN. C.BrowneJ. A.De ParkS.. (2012). Pan-genomic analysis of bovine monocyte-derived macrophage gene expression in response to in vitro infection with *Mycobacterium avium* subspecies *paratuberculosis*. Vet. Res. 43:25. doi: 10.1186/1297-9716-43-25, PMID: 22455317PMC3411445

[ref175] MageeD. A.ConlonK. M.NalpasN. C.BrowneJ. A.PirsonC.HealyC.. (2014). Innate cytokine profiling of bovine alveolar macrophages reveals commonalities and divergence in the response to *Mycobacterium bovis* and *Mycobacterium tuberculosis* infection. Tuberculosis 94, 441–450. doi: 10.1016/j.tube.2014.04.004, PMID: 24882682

[ref176] MageeD. A.TaraktsoglouM.KillickK. E.NalpasN. C.BrowneJ. A.ParkS. D. E.. (2012). Global gene expression and systems biology analysis of bovine monocyte-derived macrophages in response to in vitro challenge with *Mycobacterium bovis*. PLoS One 7:e32034. doi: 10.1371/journal.pone.0032034, PMID: 22384131PMC3284544

[ref177] MahlaR.ReddyC.PrasadD.KumarH. (2013). Sweeten PAMPs: role of sugar complexed PAMPs in innate immunity and vaccine biology. Front. Immunol. 4:248. doi: 10.3389/fimmu.2013.00248, PMID: 24032031PMC3759294

[ref178] MahonR. N.SandeO. J.RojasR. E.LevineA. D.HardingC. V.Henry BoomW. (2012). *Mycobacterium tuberculosis* ManLAM inhibits T-cell-receptor signaling by interference with ZAP-70, Lck and LAT phosphorylation. Cell. Immunol. 275, 98–105. doi: 10.1016/j.cellimm.2012.02.009, PMID: 22507872PMC3352599

[ref179] MairI.McNeillyT. N.Corripio-MiyarY.FormanR.ElseK. J. (2021). Embracing nature’s complexity: Immunoparasitology in the wild. Semin. Immunol. 53:101525. doi: 10.1016/j.smim.2021.101525, PMID: 34785137PMC8713030

[ref180] MajiA.MisraR.Kumar MondalA.KumarD.BajajD.SinghalA.. (2015). Expression profiling of lymph nodes in tuberculosis patients reveal inflammatory milieu at site of infection. Sci. Rep. 5:15214. doi: 10.1038/srep15214, PMID: 26469538PMC4606593

[ref181] MaloneK. M.Rue-AlbrechtK.MageeD. A.ConlonK.SchubertO. T.NalpasN. C.. (2018). Comparative 'omics analyses differentiate *Mycobacterium tuberculosis* and *Mycobacterium bovis* and reveal distinct macrophage responses to infection with the human and bovine tubercle bacilli. Microbial. Genomics 4:e000163. doi: 10.1099/mgen.0.000163, PMID: 29557774PMC5885015

[ref182] MancaC.TsenovaL.FreemanS.BarczakA. K.ToveyM.MurrayP. J.. (2005). Hypervirulent *M. tuberculosis* W/Beijing strains upregulate type I IFNs and increase expression of negative regulators of the Jak-Stat pathway. J. Interf. Cytokine Res. 25, 694–701. doi: 10.1089/jir.2005.25.694, PMID: 16318583

[ref183] María IreneC.-C.Juan GermánR.-C.GamalielL.-L.Dulce AdrianaM.-E.Estela IsabelB.Brenda NohemíM. C.. (2021). Profiling the immune response to *Mycobacterium tuberculosis* Beijing family infection: a perspective from the transcriptome. Virulence 12, 1689–1704. doi: 10.1080/21505594.2021.1936432, PMID: 34228582PMC8265813

[ref184] MarsayL.MatsumiyaM.TannerR.PoyntzH.GriffithsK. L.StylianouE.. (2013). Mycobacterial growth inhibition in murine splenocytes as a surrogate for protection against *Mycobacterium tuberculosis* (M. tb). Tuberculosis 93, 551–557. doi: 10.1016/j.tube.2013.04.007, PMID: 23726784

[ref185] MascarelloA.ChiaradiaL. D.VernalJ.VillarinoA.GuidoR. V. C.PerizzoloP.. (2010). Inhibition of *Mycobacterium tuberculosis* tyrosine phosphatase PtpA by synthetic chalcones: kinetics, molecular modeling, toxicity and effect on growth. Bioorg. Med. Chem. 18, 3783–3789. doi: 10.1016/j.bmc.2010.04.051, PMID: 20462762

[ref186] MasonM. J.FanG.PlathK.ZhouQ.HorvathS. (2009). Signed weighted gene co-expression network analysis of transcriptional regulation in murine embryonic stem cells. BMC Genomics 10:327. doi: 10.1186/1471-2164-10-327, PMID: 19619308PMC2727539

[ref187] McLoughlinK. E.CorreiaC. N.BrowneJ. A.MageeD. A.NalpasN. C.Rue-AlbrechtK.. (2021a). RNA-seq transcriptome analysis of peripheral blood from cattle infected with *Mycobacterium bovis* across an experimental time ccourse. Front. Vet. Sci. 8:662002. doi: 10.3389/fvets.2021.662002, PMID: 34124223PMC8193354

[ref188] McLoughlinK. E.CorreiaC. N.BrowneJ. A.MageeD. A.NalpasN. C.Rue-AlbrechtK.. (2021b). RNA-seq transcriptome analysis of peripheral blood from cattle infected with *Mycobacterium bovis* across an experimental time course. Front. Vet. Sci. 8:662002. doi: 10.3389/fvets.2021.662002, PMID: 34124223PMC8193354

[ref189] McLoughlinK. E.NalpasN. C.Rue-AlbrechtK.BrowneJ. A.MageeD. A.KillickK. E.. (2014). RNA-seq transcriptional profiling of peripheral blood leukocytes from cattle infected with *Mycobacterium bovis*. Front. Immunol. 5:396. doi: 10.3389/fimmu.2014.00396, PMID: 25206354PMC4143615

[ref190] MeadeK. G.GormleyE.DoyleM. B.FitzsimonsT.O'FarrellyC.CostelloE.. (2007). Innate gene repression associated with *Mycobacterium bovis* infection in cattle: toward a gene signature of disease. BMC Genomics 8:400. doi: 10.1186/1471-2164-8-400, PMID: 17974019PMC2213678

[ref191] MeansT. K.GolenbockD. T.FentonM. J. (2000). The biology of toll-like receptors. Cytokine Growth Factor Rev. 11, 219–232. doi: 10.1016/S1359-6101(00)00006-X10817965

[ref192] MeenuS.ThiagarajanS.RamalingamS.MichaelA.RamalingamS. (2016). Modulation of host ubiquitin system genes in human endometrial cell line infected with *Mycobacterium tuberculosis*. Med. Microbiol. Immunol. 205, 163–171. doi: 10.1007/s00430-015-0432-z, PMID: 26403675

[ref193] MeunierE.NeyrollesO. (2019). Die another way: Ferroptosis drives tuberculosis pathology. J. Exp. Med. 216, 471–473. doi: 10.1084/jem.20190038, PMID: 30787032PMC6400539

[ref194] MiaoL.YinR.-X.ZhangQ.-H.LiaoP.-J.WangY.NieR.-J.. (2019). A novel circRNA-miRNA-mRNA network identifies circ-YOD1 as a biomarker for coronary artery disease. Sci. Rep. 9:18314. doi: 10.1038/s41598-019-54603-2, PMID: 31797949PMC6892882

[ref195] MiddletonS.SteinbachS.CoadM.McGillK.BradyC.DuignanA.. (2021). A molecularly defined skin test reagent for the diagnosis of bovine tuberculosis compatible with vaccination against Johne’s disease. Sci. Rep. 11:2929. doi: 10.1038/s41598-021-82434-7, PMID: 33536465PMC7859399

[ref196] MogucheA. O.MusvosviM.Penn-NicholsonA.PlumleeC. R.MearnsH.GeldenhuysH.. (2017). Antigen availability shapes T cell differentiation and function during tuberculosis. Cell Host Microbe 21, 695–706.e5. doi: 10.1016/j.chom.2017.05.012, PMID: 28618268PMC5533182

[ref197] MoguesT.GoodrichM. E.RyanL.LaCourseR.NorthR. J. (2001). The relative importance of T cell subsets in immunity and immunopathology of airborne *Mycobacterium tuberculosis* infection in mice. J. Exp. Med. 193, 271–280. doi: 10.1084/jem.193.3.271, PMID: 11157048PMC2195922

[ref198] MohareerK.AsallaS.BanerjeeS. (2018). Cell death at the cross roads of host-pathogen interaction in *Mycobacterium tuberculosis* infection. Tuberculosis 113, 99–121. doi: 10.1016/j.tube.2018.09.007, PMID: 30514519

[ref199] MukundK.SubramaniamS. (2015). Dysregulated mechanisms underlying Duchenne muscular dystrophy from co-expression network preservation analysis. BMC. Res. Notes 8:182. doi: 10.1186/s13104-015-1141-9, PMID: 25935398PMC4424514

[ref200] NaeemM. A.AhmadW.TyagiR.AkramQ.YounusM.LiuX. (2021). Stealth strategies of *Mycobacterium tuberculosis* for immune evasion. Curr. Issues Mol. Biol. 41, 597–616. doi: 10.21775/cimb.041.597, PMID: 33068079

[ref201] NagabhushanamV.SolacheA.TingL.-M.EscaronC. J.ZhangJ. Y.ErnstJ. D. (2003). Innate inhibition of adaptive immunity: *Mycobacterium tuberculosis*-induced IL6 inhibits macrophage responses to IFN-γ. J. Immunol. 171, 4750–4757. doi: 10.4049/jimmunol.171.9.4750, PMID: 14568951

[ref202] NagerM.TarrP. E.HaackH. G.MartiusF.StoebeC.FreiR.. (2009). Reactivation of bovine tuberculosis in patient treated with infliximab, Switzerland. Emerg. Infect. Dis. J. 15:1132, –1133. doi: 10.3201/eid1507.090024, PMID: 19624941PMC2744244

[ref203] NalpasN. C.MageeD. A.ConlonK. M.BrowneJ. A.HealyC.McLoughlinK. E.. (2015). RNA sequencing provides exquisite insight into the manipulation of the alveolar macrophage by tubercle bacilli. Sci. Rep. 5:13629. doi: 10.1038/srep13629, PMID: 26346536PMC4642568

[ref204] NalpasN. C.ParkS. D. E.MageeD. A.TaraktsoglouM.BrowneJ. A.ConlonK. M.. (2013). Whole-transcriptome, high-throughput RNA sequence analysis of the bovine macrophage response to *Mycobacterium bovis* infection in vitro. BMC Genomics 14:230. doi: 10.1186/1471-2164-14-230, PMID: 23565803PMC3640917

[ref206] NdlovuH.MarakalalaM. J. (2016). Granulomas and inflammation: host-directed therapies for tuberculosis. Front. Immunol. 7:434. doi: 10.3389/fimmu.2016.00434, PMID: 27822210PMC5075764

[ref207] NeteaM. G.Van der MeerJ. W. M.KullbergB.-J. (2004). Toll-like receptors as an escape mechanism from the host defense. Trends Microbiol. 12, 484–488. doi: 10.1016/j.tim.2004.09.004, PMID: 15488388

[ref208] Ní CheallaighC.KeaneJ.LavelleE. C.HopeJ. C.HarrisJ. (2011). Autophagy in the immune response to tuberculosis: clinical perspectives. Clin. Exp. Immunol. 164, 291–300. doi: 10.1111/j.1365-2249.2011.04381.x, PMID: 21438870PMC3087924

[ref209] NossE. H.PaiR. K.SellatiT. J.RadolfJ. D.BelisleJ.GolenbockD. T.. (2001). Toll-like receptor 2-dependent inhibition of macrophage class II MHC expression and antigen processing by 19-kDa lipoprotein of *Mycobacterium tuberculosis*. J. Immunol. 167, 910–918. doi: 10.4049/jimmunol.167.2.910, PMID: 11441098

[ref210] NougayrèdeJ.-P.TaiebF.RyckeJ. D.OswaldE. (2005). Cyclomodulins: bacterial effectors that modulate the eukaryotic cell cycle. Trends Microbiol. 13, 103–110. doi: 10.1016/j.tim.2005.01.002, PMID: 15737728

[ref211] Olea-PopelkaF.MuwongeA.PereraA.DeanA. S.MumfordE.Erlacher-VindelE.. (2017). Zoonotic tuberculosis in human beings caused by *Mycobacterium bovis*—a call for action. Lancet Infect. Dis. 17, e21–e25. doi: 10.1016/S1473-3099(16)30139-6, PMID: 27697390

[ref212] O'LearyS.O'SullivanM. P.KeaneJ. (2011). IL-10 blocks phagosome maturation in *Mycobacterium tuberculosis*–infected human macrophages. Am. J. Respir. Cell Mol. Biol. 45, 172–180. doi: 10.1165/rcmb.2010-0319OC, PMID: 20889800

[ref213] PadhiA.PattnaikK.BiswasM.JagadebM.BeheraA.SonawaneA. (2019). *Mycobacterium tuberculosis* LprE suppresses TLR2-dependent cathelicidin and autophagy expression to enhance bacterial survival in macrophages. J. Immunol. 203, 2665–2678. doi: 10.4049/jimmunol.1801301, PMID: 31619537

[ref214] PahariS.KaurG.AqdasM.NegiS.ChatterjeeD.BashirH.. (2017). Bolstering immunity through pattern recognition receptors: A unique approach to control tuberculosis. Front. Immunol. 8:906. doi: 10.3389/fimmu.2017.00906, PMID: 28824632PMC5539433

[ref215] PaikS.KimJ. K.ChungC.JoE.-K. (2019). Autophagy: A new strategy for host-directed therapy of tuberculosis. Virulence 10, 448–459. doi: 10.1080/21505594.2018.1536598, PMID: 30322337PMC6550549

[ref216] PajueloD.Gonzalez-JuarbeN.NiederweisM. (2020). NAD hydrolysis by the tuberculosis necrotizing toxin induces lethal oxidative stress in macrophages. Cell. Microbiol. 22:e13115. doi: 10.1111/cmi.13115, PMID: 31509891PMC6925628

[ref217] PalmerM. V.ThackerT. C.RabideauM. M.JonesG. J.KanipeC.VordermeierH. M.. (2020). Biomarkers of cell-mediated immunity to bovine tuberculosis. Vet. Immunol. Immunopathol. 220:109988. doi: 10.1016/j.vetimm.2019.109988, PMID: 31846797

[ref218] PappA. C.AzadA. K.PietrzakM.WilliamsA.HandelmanS. K.IgoR. P.Jr.. (2018). AmpliSeq transcriptome analysis of human alveolar and monocyte-derived macrophages over time in response to *Mycobacterium tuberculosis* infection. PLoS One 13:e0198221. doi: 10.1371/journal.pone.0198221, PMID: 29847580PMC5976201

[ref219] ParasaV. R.MuvvaJ. R.RoseJ. F.BraianC.BrighentiS.LermM. (2017). Inhibition of tissue matrix metalloproteinases interferes with *Mycobacterium tuberculosis*-induced granuloma formation and reduces bacterial load in a human lung tissue model. Front. Microbiol. 8:2370. doi: 10.3389/fmicb.2017.02370, PMID: 29259583PMC5723394

[ref220] ParkS. K.ParkC.-S.LeeH.-S.ParkK. S.ParkB. L.CheongH. S.. (2014). Functional polymorphism in aldehyde dehydrogenase-2 gene associated with risk of tuberculosis. BMC Med. Genet. 15:40. doi: 10.1186/1471-2350-15-40, PMID: 24690209PMC3975138

[ref221] PathakS. K.BasuS.BasuK. K.BanerjeeA.PathakS.BhattacharyyaA.. (2007). Direct extracellular interaction between the early secreted antigen ESAT-6 of *Mycobacterium tuberculosis* and TLR2 inhibits TLR signaling in macrophages. Nat. Immunol. 8, 610–618. doi: 10.1038/ni1468, PMID: 17486091

[ref222] PawarK.SharbatiJ.EinspanierR.SharbatiS. (2016). *Mycobacterium bovis* BCG interferes with miR-3619-5p control of cathepsin S in the process of autophagy. Front. Cell. Infect. Microbiol. 6:27. doi: 10.3389/fcimb.2016.00027, PMID: 27014637PMC4783571

[ref223] PetrilliJ. D.AraújoL. E.da SilvaL. S.LausA. C.MüllerI.ReisR. M.. (2020). Whole blood mRNA expression-based targets to discriminate active tuberculosis from latent infection and other pulmonary diseases. Sci. Rep. 10:22072. doi: 10.1038/s41598-020-78793-2, PMID: 33328540PMC7745039

[ref224] PiercyJ.WerlingD.CoffeyT. J. (2007). Differential responses of bovine macrophages to infection with bovine-specific and non-bovine specific mycobacteria. Tuberculosis 87, 415–420. doi: 10.1016/j.tube.2007.06.001, PMID: 17644438

[ref225] PiresD.BernardE. M.PomboJ. P.CarmoN.FialhoC.GutierrezM. G.. (2017). *Mycobacterium tuberculosis* modulates miR-106b-5p to control cathepsin S expression resulting in higher pathogen survival and poor T-cell activation. Front. Immunol. 8:1819. doi: 10.3389/fimmu.2017.01819, PMID: 29326705PMC5741618

[ref227] PlacidoR.MancinoG.AmendolaA.MarianiF.VendettiS.PiacentiniM.. (1997). Apoptosis of human monocytes/macrophages in *Mycobacterium tuberculosis* infection. J. Pathol. 181, 31–38. doi: 10.1002/(SICI)1096-9896(199701)181:1<31::AID-PATH722>3.0.CO;2-G, PMID: 9072000

[ref228] PollockJ. M.NeillS. D. (2002). *Mycobacterium bovis* infection and tuberculosis in cattle. Vet. J. 163, 115–127. doi: 10.1053/tvjl.2001.065512093187

[ref229] PollockJ. M.PollockD. A.CampbellD. G.GirvinR. M.CrockardA. D.NeillS. D.. (1996). Dynamic changes in circulating and antigen-responsive T-cell subpopulations post-*Mycobacterium bovis* infection in cattle. Immunology 87, 236–241. doi: 10.1046/j.1365-2567.1996.457538.x, PMID: 8698385PMC1384279

[ref230] PollockJ. M.RodgersJ. D.WelshM. D.McNairJ. (2006). Pathogenesis of bovine tuberculosis: the role of experimental models of infection. Vet. Microbiol. 112, 141–150. doi: 10.1016/j.vetmic.2005.11.03216384665

[ref231] QuallsJ. E.MurrayP. J. (2016). Immunometabolism within the tuberculosis granuloma: amino acids, hypoxia, and cellular respiration. Semin. Immunopathol. 38, 139–152. doi: 10.1007/s00281-015-0534-0, PMID: 26490974PMC4779414

[ref232] Quesnel-VallièresM.WeatherittR. J.CordesS. P.BlencoweB. J. (2019). Autism spectrum disorder: insights into convergent mechanisms from transcriptomics. Nat. Rev. Genet. 20, 51–63. doi: 10.1038/s41576-018-0066-2, PMID: 30390048

[ref233] Riquelme MedinaI.Lubovac-PilavZ. (2016). Gene co-expression network analysis for identifying modules and functionally enriched pathways in type 1 diabetes. PLoS One 11:e0156006. doi: 10.1371/journal.pone.0156006, PMID: 27257970PMC4892488

[ref234] Rivero-LezcanoO. M.González-CortésC.Reyes-RuvalcabaD.Diez-TascónC. (2010). CCL20 is overexpressed in *Mycobacterium tuberculosis*-infected monocytes and inhibits the production of reactive oxygen species (ROS). Clin. Exp. Immunol. 162, 289–297. doi: 10.1111/j.1365-2249.2010.04168.x, PMID: 20819093PMC2996596

[ref236] RohdeK.YatesR. M.PurdyG. E.RussellD. G. (2007). *Mycobacterium tuberculosis* and the environment within the phagosome. Immunol. Rev. 219, 37–54. doi: 10.1111/j.1600-065X.2007.00547.x17850480

[ref237] RojasM.BarreraL. F.GarcíaL. F. (1998). Induction of apoptosis in murine macrophages by *Mycobacterium tuberculosis* is reactive oxygen intermediates-independent. Biochem. Biophys. Res. Commun. 247, 436–442. doi: 10.1006/bbrc.1998.8802, PMID: 9642146

[ref238] RoyA.Díez-GuerrierA.OrtegaJ.de la CruzM. L.SáezJ. L.DomínguezL.. (2019). Evaluation of the McLintock syringe as a cause of non-specific reactions in the intradermal tuberculin test used for the diagnosis of bovine tuberculosis. Res. Vet. Sci. 122, 175–178. doi: 10.1016/j.rvsc.2018.11.025, PMID: 30529272

[ref239] RuskR. A.PalmerM. V.WatersW. R.McGillJ. L. (2017). Measuring bovine γδ T cell function at the site of *Mycobacterium bovis* infection. Vet. Immunol. Immunopathol. 193–194, 38–49. doi: 10.1016/j.vetimm.2017.10.004, PMID: 29129226PMC5703227

[ref240] RussellD. G.CardonaP.-J.KimM.-J.AllainS.AltareF. (2009). Foamy macrophages and the progression of the human tuberculosis granuloma. Nat. Immunol. 10, 943–948. doi: 10.1038/ni.1781, PMID: 19692995PMC2759071

[ref241] Sabio y GarcíaJ.BigiM. M.KleppL. I.GarcíaE. A.BlancoF. C.BigiF. (2020). Does *Mycobacterium bovis* persist in cattle in a non-replicative latent state as *Mycobacterium tuberculosis* in human beings? Vet. Microbiol. 247:108758. doi: 10.1016/j.vetmic.2020.108758, PMID: 32768211

[ref242] SakowskiE. T.KosterS.Portal CelhayC.ParkH. S.ShresthaE.HetzeneckerS. E.. (2015). Ubiquilin 1 promotes IFN-γ-induced xenophagy of *Mycobacterium tuberculosis*. PLoS Pathog. 11:e1005076. doi: 10.1371/journal.ppat.1005076, PMID: 26225865PMC4520715

[ref243] SalgameP. (2005). Host innate and Th1 responses and the bacterial factors that control *Mycobacterium tuberculosis* infection. Curr. Opin. Immunol. 17, 374–380. doi: 10.1016/j.coi.2005.06.006, PMID: 15963709

[ref244] SalgameP. (2011). MMPs in tuberculosis: granuloma creators and tissue destroyers. J. Clin. Invest. 121, 1686–1688. doi: 10.1172/JCI57423, PMID: 21519148PMC3083780

[ref245] SambareyA.DevaprasadA.BaloniP.MishraM.MohanA.TyagiP.. (2017). Meta-analysis of host response networks identifies a common core in tuberculosis. NPJ Syst. Biol. Appl. 3:4. doi: 10.1038/s41540-017-0005-4, PMID: 28649431PMC5445610

[ref246] SamtenB.WangX.BarnesP. F. (2009). *Mycobacterium tuberculosis* ESX-1 system-secreted protein ESAT-6 but not CFP10 inhibits human T-cell immune responses. Tuberculosis 89, S74–S76. doi: 10.1016/S1472-9792(09)70017-4, PMID: 20006311

[ref247] Sánchez-SotoE.Ponce-RamosR.Hernández-GutiérrezR.Gutiérrez-OrtegaA.ÁlvarezA. H.Martínez-VelázquezM.. (2017). Colostrum proinflammatory cytokines as biomarkers of bovine immune response to bovine tuberculosis (bTB). Microb. Pathog. 103, 57–64. doi: 10.1016/j.micpath.2016.12.007, PMID: 28007592

[ref248] SandeO. J.KarimA. F.LiQ.DingX.HardingC. V.RojasR. E.. (2016). Mannose-capped lipoarabinomannan from *Mycobacterium tuberculosis* induces CD4+ T cell anergy *via* GRAIL. J. Immunol. 196, 691–702. doi: 10.4049/jimmunol.1500710, PMID: 26667170PMC4707121

[ref249] SchaaleK.NeumannJ.SchneiderD.EhlersS.ReilingN. (2011). Wnt signaling in macrophages: augmenting and inhibiting mycobacteria-induced inflammatory responses. Eur. J. Cell Biol. 90, 553–559. doi: 10.1016/j.ejcb.2010.11.004, PMID: 21185106

[ref250] SchillerI.OeschB.VordermeierH. M.PalmerM. V.HarrisB. N.OrloskiK. A.. (2010). Bovine tuberculosis: A review of current and emerging diagnostic techniques in view of their relevance for disease control and eradication. Transbound. Emerg. Dis. 57, 205–220. doi: 10.1111/j.1865-1682.2010.01148.x, PMID: 20561288

[ref251] SchneiderH.DowneyJ.SmithA.ZinselmeyerB. H.RushC.BrewerJ. M.. (2006). Reversal of the TCR stop signal by CTLA-4. Science 313, 1972–1975. doi: 10.1126/science.1131078, PMID: 16931720

[ref253] SetoS.MorimotoK.YoshidaT.HiramatsuM.HijikataM.NagataT.. (2020). Proteomic profiling reveals the architecture of granulomatous lesions caused by tuberculosis and *Mycobacterium avium* complex lung disease. Front. Microbiol. 10:3081. doi: 10.3389/fmicb.2019.03081, PMID: 32010116PMC6978656

[ref254] ShapiraT.Rankine-WilsonL.ChaoJ. D.PichlerV.RensC.PfeiferT.. (2020). High-content screening of eukaryotic kinase inhibitors identify CHK2 inhibitor activity against *Mycobacterium tuberculosis*. Front. Microbiol. 11:553962. doi: 10.3389/fmicb.2020.553962, PMID: 33042061PMC7530171

[ref255] SharifiS.PakdelA.EbrahimieE.AryanY.Ghaderi ZefreheeM.ReecyJ. M. (2019). Prediction of key regulators and downstream targets of E. coli induced mastitis. J. Appl. Genet. 60, 367–373. doi: 10.1007/s13353-019-00499-7, PMID: 31187384

[ref256] ShariqM.QuadirN.SharmaN.SinghJ.SheikhJ. A.KhubaibM.. (2021). *Mycobacterium tuberculosis* RipA dampens TLR4-mediated host protective response using a multi-pronged approach involving autophagy, apoptosis, metabolic repurposing, and immune modulation. Front. Immunol. 12:636644. doi: 10.3389/fimmu.2021.636644, PMID: 33746976PMC7969667

[ref257] SharmaS.RyndakM. B.AggarwalA. N.YadavR.SethiS.MasihS.. (2017). Transcriptome analysis of mycobacteria in sputum samples of pulmonary tuberculosis patients. PLoS One 12:e0173508. doi: 10.1371/journal.pone.0173508, PMID: 28282458PMC5345810

[ref258] SharmaM.SharmaS.RoyS.VarmaS.BoseM. (2007). Pulmonary epithelial cells are a source of interferon-γ in response to *Mycobacterium tuberculosis* infection. Immunol. Cell Biol. 85, 229–237. doi: 10.1038/sj.icb.7100037, PMID: 17310225

[ref259] SharmaG.SowpatiD. T.SinghP.KhanM. Z.GanjiR.UpadhyayS.. (2016). Genome-wide non-CpG methylation of the host genome during *M. tuberculosis* infection. Sci. Rep. 6:25006. doi: 10.1038/srep25006, PMID: 27112593PMC4845000

[ref260] SheridanM. P.BrowneJ. A.DoyleM. B.FitzsimonsT.McGillK.GormleyE. (2017). IL-10 suppression of IFN-γ responses in tuberculin-stimulated whole blood from *Mycobacterium bovis* infected cattle. Vet. Immunol. Immunopathol. 189, 36–42. doi: 10.1016/j.vetimm.2017.06.003, PMID: 28669385

[ref261] SheybaniN.BakhtiarizadehM. R.SalehiA. (2021). An integrated analysis of mRNAs, lncRNAs, and miRNAs based on weighted gene co-expression network analysis involved in bovine endometritis. Sci. Rep. 11:18050. doi: 10.1038/s41598-021-97319-y, PMID: 34508138PMC8433134

[ref262] ShiL.SalamonH.EugeninE. A.PineR.CooperA.GennaroM. L. (2015). Infection with *Mycobacterium tuberculosis* induces the Warburg effect in mouse lungs. Sci. Rep. 5:18176. doi: 10.1038/srep18176, PMID: 26658723PMC4674750

[ref263] ShiL.WenZ.LiH.SongY. (2021). Identification of hub genes associated with tuberculous pleurisy by integrated bioinformatics analysis. Front. Genet. 12:730491. doi: 10.3389/fgene.2021.730491, PMID: 34925441PMC8678451

[ref264] ShuklaS. K.ShuklaS.ChauhanA.SarvjeetKhanR.AhujaA.. (2017). Differential gene expression in *Mycobacterium bovis* challenged monocyte-derived macrophages of cattle. Microb. Pathog. 113, 480–489. doi: 10.1016/j.micpath.2017.11.030, PMID: 29170044

[ref265] ShuklaS. K.ShuklaS.KhanR.AhujaA.SinghL. V.KambleN. M.. (2018). Pathway analysis of differentially expressed genes in *Mycobacterium bovis* challenged bovine macrophages. Microb. Pathog. 115, 343–352. doi: 10.1016/j.micpath.2017.11.065, PMID: 29197526

[ref266] SilvaC. A.Ribeiro-dos-SantosA.GonçalvesW. G.PintoP.PantojaR. P.Vinasco-SandovalT.. (2021). Can miRNA indicate risk of illness after continuous exposure to *M. tuberculosis*? Int. J. Mol. Sci. 22:3674. doi: 10.3390/ijms22073674, PMID: 33916069PMC8036329

[ref267] Silveira-MattosP. S.Barreto-DuarteB.VasconcelosB.FukutaniK. F.VinhaesC. L.Oliveira-De-SouzaD.. (2019). Differential expression of activation markers by *Mycobacterium tuberculosis*-specific CD4+ T cell distinguishes extrapulmonary from pulmonary tuberculosis and latent infection. Clin. Infect. Dis. 71, 1905–1911. doi: 10.1093/cid/ciz1070, PMID: 31665254PMC8463092

[ref268] SimmonsD. P.CanadayD. H.LiuY.LiQ.HuangA.BoomW. H.. (2010). *Mycobacterium tuberculosis* and TLR2 agonists inhibit induction of type I IFN and class I MHC antigen cross processing by TLR9. J. Immunol. 185, 2405–2415. doi: 10.4049/jimmunol.0904005, PMID: 20660347PMC2990778

[ref269] SkinnerM. A.ParlaneN.McCarthyA.BuddleB. M. (2003). Cytotoxic T-cell responses to *Mycobacterium bovis* during experimental infection of cattle with bovine tuberculosis. Immunology 110, 234–241. doi: 10.1046/j.1365-2567.2003.01731.x, PMID: 14511237PMC1783035

[ref270] SmithN. H.GordonS. V.de la Rua-DomenechR.Clifton-HadleyR. S.HewinsonR. G. (2006). Bottlenecks and broomsticks: the molecular evolution of *Mycobacterium bovis*. Nat. Rev. Microbiol. 4, 670–681. doi: 10.1038/nrmicro1472, PMID: 16912712

[ref271] SmythG. K. (2005). “Limma: linear models for microarray data” in Bioinformatics and Computational Biology Solutions Using R and Bioconductor. eds. GentlemanR.CareyV. J.HuberW.IrizarryR. A.DudoitS. (New York, NY: Springer New York), 397–420.

[ref272] SongL.LangfelderP.HorvathS. (2012). Comparison of co-expression measures: mutual information, correlation, and model based indices. BMC Bioinf. 13:328. doi: 10.1186/1471-2105-13-328, PMID: 23217028PMC3586947

[ref273] SonganeM.KleinnijenhuisJ.NeteaM. G.van CrevelR. (2012). The role of autophagy in host defence against *Mycobacterium tuberculosis* infection. Tuberculosis 92, 388–396. doi: 10.1016/j.tube.2012.05.004, PMID: 22683183

[ref274] StrongE. J.WangJ.NgT. W.PorcelliS. A.LeeS.SiegristM. S. (2022). *Mycobacterium tuberculosis* PPE51 inhibits autophagy by suppressing toll-like receptor 2-dependent signaling. MBio 13, e02974–e02921. doi: 10.1128/mbio.02974-21, PMID: 35467412PMC9239179

[ref275] SubuddhiA.KumarM.MajumderD.SarkarA.GhoshZ.VasudevanM.. (2020). Unraveling the role of H3K4 trimethylation and lncRNA HOTAIR in SATB1 and DUSP4-dependent survival of virulent *Mycobacterium tuberculosis* in macrophages. Tuberculosis 120:101897. doi: 10.1016/j.tube.2019.101897, PMID: 32090865

[ref276] SunY.ChenG.LiuZ.YuL.ShangY. (2020). A bioinformatics analysis to identify novel biomarkers for prognosis of pulmonary tuberculosis. BMC Pulm. Med. 20:279. doi: 10.1186/s12890-020-01316-2, PMID: 33099324PMC7585184

[ref277] SzklarczykD.GableA. L.LyonD.JungeA.WyderS.Huerta-CepasJ.. (2018). STRING v11: protein–protein association networks with increased coverage, supporting functional discovery in genome-wide experimental datasets. Nucleic Acids Res. 47, D607–D613. doi: 10.1093/nar/gky1131, PMID: 30476243PMC6323986

[ref278] TangD.KangR.CoyneC. B.ZehH. J.LotzeM. T. (2012). PAMPs and DAMPs: signal 0s that spur autophagy and immunity. Immunol. Rev. 249, 158–175. doi: 10.1111/j.1600-065X.2012.01146.x, PMID: 22889221PMC3662247

[ref279] ThakurA.AndreaA.MikkelsenH.WoodworthJ. S.AndersenP.JungersenG.. (2018). Targeting the Mincle and TLR3 receptor using the dual agonist cationic adjuvant formulation 9 (CAF09) induces humoral and polyfunctional memory T cell responses in calves. PLoS One 13:e0201253. doi: 10.1371/journal.pone.0201253, PMID: 30063728PMC6067743

[ref280] TrinchieriG.SherA. (2007). Cooperation of toll-like receptor signals in innate immune defence. Nat. Rev. Immunol. 7, 179–190. doi: 10.1038/nri2038, PMID: 17318230

[ref281] TripathiD.WelchE.CheekatlaS. S.RadhakrishnanR. K.VenkatasubramanianS.PaidipallyP.. (2018). Alcohol enhances type 1 interferon-α production and mortality in young mice infected with *Mycobacterium tuberculosis*. PLoS Pathog. 14:e1007174. doi: 10.1371/journal.ppat.1007174, PMID: 30071107PMC6072099

[ref282] TsaiK.-N.ChanE.-C.TsaiT.-Y.ChenK.-T.ChenC.-Y.HungK.. (2009). Cytotoxic effect of recombinant *Mycobacterium tuberculosis* CFP-10/ESAT-6 protein on the crucial pathways of WI-38 cells. J. Biomed. Biotechnol. 2009:917084. doi: 10.1155/2009/917084, PMID: 19584916PMC2702506

[ref283] VainchenkerW.ConstantinescuS. N. (2013). JAK/STAT signaling in hematological malignancies. Oncogene 32, 2601–2613. doi: 10.1038/onc.2012.34722869151

[ref284] van DamS.VõsaU.van der GraafA.FrankeL.de MagalhãesJ. P. (2017). Gene co-expression analysis for functional classification and gene–disease predictions. Brief. Bioinform. 19, bbw139–bbw592. doi: 10.1093/bib/bbw139, PMID: 28077403PMC6054162

[ref285] VayrF.Martin-BlondelG.SavallF.SoulatJ.-M.DeffontainesG.HerinF. (2018). Occupational exposure to human *Mycobacterium bovis* infection: A systematic review. PLoS Negl. Trop. Dis. 12:e0006208. doi: 10.1371/journal.pntd.0006208, PMID: 29337996PMC5786333

[ref286] Vega-ManriquezX.López-VidalY.MoranJ.AdamsL. G.Gutiérrez-PabelloJ. A. (2007). Apoptosis-inducing factor participation in bovine macrophage *Mycobacterium bovis*-induced caspase-independent cell death. Infect. Immun. 75, 1223–1228. doi: 10.1128/IAI.01047-06, PMID: 17158896PMC1828566

[ref287] VeghP.MageeD. A.NalpasN. C.BryanK.McCabeM. S.BrowneJ. A.. (2015). MicroRNA profiling of the bovine alveolar macrophage response to *Mycobacterium bovis* infection suggests pathogen survival is enhanced by microRNA regulation of endocytosis and lysosome trafficking. Tuberculosis 95, 60–67. doi: 10.1016/j.tube.2014.10.011, PMID: 25692199

[ref288] VereeckeL.BeyaertR.van LooG. (2009). The ubiquitin-editing enzyme A20 (TNFAIP3) is a central regulator of immunopathology. Trends Immunol. 30, 383–391. doi: 10.1016/j.it.2009.05.007, PMID: 19643665

[ref289] VillarinoA. V.KannoY.O'SheaJ. J. (2017). Mechanisms and consequences of Jak–STAT signaling in the immune system. Nat. Immunol. 18, 374–384. doi: 10.1038/ni.3691, PMID: 28323260PMC11565648

[ref290] Villarreal-RamosB.BergS.WhelanA.HolbertS.CarrerasF.SalgueroF. J.. (2018). Experimental infection of cattle with *Mycobacterium tuberculosis* isolates shows the attenuation of the human tubercle bacillus for cattle. Sci. Rep. 8:894. doi: 10.1038/s41598-017-18575-5, PMID: 29343690PMC5772528

[ref291] VinayagamA.GibsonT. E.LeeH.-J.YilmazelB.RoeselC.HuY.. (2016). Controllability analysis of the directed human protein interaction network identifies disease genes and drug targets. Proc. Natl. Acad. Sci. 113, 4976–4981. doi: 10.1073/pnas.1603992113, PMID: 27091990PMC4983807

[ref292] VordermeierH. M.ChambersM. A.CockleP. J.WhelanA. O.SimmonsJ.HewinsonR. G. (2002). Correlation of ESAT-6-specific gamma interferon production with pathology in cattle following *Mycobacterium bovis* BCG vaccination against experimental bovine tuberculosis. Infect. Immun. 70, 3026–3032. doi: 10.1128/IAI.70.6.3026-3032.2002, PMID: 12010994PMC128013

[ref293] WalzlG.RonacherK.HanekomW.ScribaT. J.ZumlaA. (2011). Immunological biomarkers of tuberculosis. Nat. Rev. Immunol. 11, 343–354. doi: 10.1038/nri296021475309

[ref294] WanQ.TangJ.HanY.WangD. (2018). Co-expression modules construction by WGCNA and identify potential prognostic markers of uveal melanoma. Exp. Eye Res. 166, 13–20. doi: 10.1016/j.exer.2017.10.007, PMID: 29031853

[ref295] WangZ.AratS.Magid-SlavM.BrownJ. R. (2018). Meta-analysis of human gene expression in response to *Mycobacterium tuberculosis* infection reveals potential therapeutic targets. BMC Syst. Biol. 12:3. doi: 10.1186/s12918-017-0524-z, PMID: 29321020PMC5763539

[ref296] WangJ.HussainT.YueR.LiaoY.LiQ.YaoJ.. (2018). MicroRNA-199a inhibits cellular autophagy and downregulates IFN-β expression by targeting TBK1 in *Mycobacterium bovis* infected cells. Front. Cell. Infect. Microbiol. 8:238. doi: 10.3389/fcimb.2018.00238, PMID: 30042930PMC6048223

[ref297] WangL.-X.LiY.ChenG.-Z. (2018). Network-based co-expression analysis for exploring the potential diagnostic biomarkers of metastatic melanoma. PLoS One 13:e0190447. doi: 10.1371/journal.pone.0190447, PMID: 29377892PMC5788335

[ref298] WangJ.LiB.-X.GeP.-P.LiJ.WangQ.GaoG. F.. (2015). *Mycobacterium tuberculosis* suppresses innate immunity by coopting the host ubiquitin system. Nat. Immunol. 16, 237–245. doi: 10.1038/ni.3096, PMID: 25642820

[ref299] WangC.LiY.-Y.LiX.WeiL.-L.YangX.-Y.XuD.-D.. (2014). Serum complement C4b, fibronectin, and prolidase are associated with the pathological changes of pulmonary tuberculosis. BMC Infect. Dis. 14:52. doi: 10.1186/1471-2334-14-52, PMID: 24484408PMC3913605

[ref300] WangX.MehraS.KaushalD.VeazeyR. S.XuH. (2021). Abnormal tryptophan metabolism in HIV and *Mycobacterium tuberculosis* infection. Front. Microbiol. 12:666227. doi: 10.3389/fmicb.2021.666227, PMID: 34262540PMC8273495

[ref301] WangY.WangJ.TangQ.RenG. (2021). Identification of UBE2C as hub gene in driving prostate cancer by integrated bioinformatics analysis. PLoS One 16:e0247827. doi: 10.1371/journal.pone.0247827, PMID: 33630978PMC7906463

[ref302] WangY.ZhouX.LinJ.YinF.XuL.HuangY.. (2011). Effects of *Mycobacterium bovis* on monocyte-derived macrophages from bovine tuberculosis infection and healthy cattle. FEMS Microbiol. Lett. 321, 30–36. doi: 10.1111/j.1574-6968.2011.02304.x, PMID: 21569079

[ref303] WangJ.ZhouX.PanB.WangH.ShiF.GanW.. (2013). Expression pattern of interferon-inducible transcriptional genes in neutrophils during bovine tuberculosis infection. DNA Cell Biol. 32, 480–486. doi: 10.1089/dna.2012.1941, PMID: 23808561

[ref304] WatersW. R.MaggioliM. F.McGillJ. L.LyashchenkoK. P.PalmerM. V. (2014). Relevance of bovine tuberculosis research to the understanding of human disease: historical perspectives, approaches, and immunologic mechanisms. Vet. Immunol. Immunopathol. 159, 113–132. doi: 10.1016/j.vetimm.2014.02.009, PMID: 24636301

[ref305] WatersW. R.PalmerM. V.BuddleB. M.VordermeierH. M. (2012). Bovine tuberculosis vaccine research: historical perspectives and recent advances. Vaccine 30, 2611–2622. doi: 10.1016/j.vaccine.2012.02.018, PMID: 22342705

[ref306] WedlockD. N.DenisM.PainterG. F.AingeG. D.VordermeierH. M.HewinsonR. G.. (2008). Enhanced protection against bovine tuberculosis after coadministration of *Mycobacterium bovis* BCG with a mycobacterial protein vaccine-adjuvant combination but not after coadministration of adjuvant alone. Clin. Vaccine Immunol. 15, 765–772. doi: 10.1128/CVI.00034-08, PMID: 18337375PMC2394838

[ref307] WeiS.-N.ZhaoW.-J.ZengX.-J.KangY.-M.DuJ.LiH.-H. (2015). Microarray and co-expression network analysis of genes associated with acute doxorubicin cardiomyopathy in mice. Cardiovasc. Toxicol. 15, 377–393. doi: 10.1007/s12012-014-9306-7, PMID: 25575753

[ref308] WeinerJ.3rdParidaS. K.MaertzdorfJ.BlackG. F.RepsilberD.TelaarA.. (2012). Biomarkers of inflammation, immunosuppression and stress are revealed by metabolomic profiling of tuberculosis patients. PLoS One 7:e40221. doi: 10.1371/journal.pone.0040221, PMID: 22844400PMC3402490

[ref309] WhiteM. J.HeH.PenoskeR. M.TwiningS. S.ZahrtT. C. (2010). PepD participates in the mycobacterial stress response mediated through MprAB and SigE. J. Bacteriol. 192, 1498–1510. doi: 10.1128/JB.01167-09, PMID: 20061478PMC2832534

[ref310] WiardaJ. E.BoggiattoP. M.BaylesD. O.WatersW. R.ThackerT. C.PalmerM. V. (2020). Severity of bovine tuberculosis is associated with innate immune-biased transcriptional signatures of whole blood in early weeks after experimental *Mycobacterium bovis* infection. PLoS One 15:e0239938. doi: 10.1371/journal.pone.0239938, PMID: 33166313PMC7652326

[ref311] WiddisonS.CoffeyT. J. (2011). Cattle and chemokines: evidence for species-specific evolution of the bovine chemokine system. Anim. Genet. 42, 341–353. doi: 10.1111/j.1365-2052.2011.02200.x, PMID: 21749416

[ref312] WiddisonS.WatsonM.CoffeyT. J. (2009). Correlation between lymph node pathology and chemokine expression during bovine tuberculosis. Tuberculosis 89, 417–422. doi: 10.1016/j.tube.2009.09.003, PMID: 19926028

[ref313] WiddisonS.WatsonM.CoffeyT. J. (2011). Early response of bovine alveolar macrophages to infection with live and heat-killed *Mycobacterium bovis*. Dev. Comp. Immunol. 35, 580–591. doi: 10.1016/j.dci.2011.01.001, PMID: 21232552

[ref314] WiddisonS.WatsonM.PiercyJ.HowardC.CoffeyT. J. (2008). Granulocyte chemotactic properties of *M. tuberculosis* versus *M. bovis*-infected bovine alveolar macrophages. Mol. Immunol. 45, 740–749. doi: 10.1016/j.molimm.2007.06.357, PMID: 17698194

[ref315] WilburnK. M.FiewegerR. A.VanderVenB. C. (2018). Cholesterol and fatty acids grease the wheels of *Mycobacterium tuberculosis* pathogenesis. Pathog. Dis. 76:fty021. doi: 10.1093/femspd/fty021, PMID: 29718271PMC6251666

[ref316] WongD.BachH.SunJ.HmamaZ.Av-GayY. (2011). *Mycobacterium tuberculosis* protein tyrosine phosphatase (PtpA) excludes host vacuolar-H+–ATPase to inhibit phagosome acidification. Proc. Natl. Acad. Sci. 108, 19371–19376. doi: 10.1073/pnas.1109201108, PMID: 22087003PMC3228452

[ref317] WongD.ChaoJ. D.Av-GayY. (2013). *Mycobacterium tuberculosis*-secreted phosphatases: from pathogenesis to targets for TB drug development. Trends Microbiol. 21, 100–109. doi: 10.1016/j.tim.2012.09.002, PMID: 23084287

[ref318] WongK.-W.JacobsW. R.Jr. (2011). Critical role for NLRP3 in necrotic death triggered by *Mycobacterium tuberculosis*. Cell. Microbiol. 13, 1371–1384. doi: 10.1111/j.1462-5822.2011.01625.x, PMID: 21740493PMC3257557

[ref319] WuS.WangM.-G.WangY.HeJ.-Q. (2019). Polymorphisms of cytokine genes and tuberculosis in two independent studies. Sci. Rep. 9:2507. doi: 10.1038/s41598-019-39249-4, PMID: 30792445PMC6385216

[ref320] WuS.WangY.ZhangM.ShresthaS. S.WangM.HeJ.-Q. (2018). Genetic polymorphisms of IL1B, IL6, and TNFα in a Chinese Han population with pulmonary tuberculosis. Biomed. Res. Int. 2018:3010898. doi: 10.1155/2018/3010898, PMID: 29888256PMC5977055

[ref321] XausJ.BesalduchN.ComaladaM.MarcovalJ.PujolR.MañáJ.. (2003). High expression of p21Waf1 in sarcoid granulomas: a putative role for long-lasting inflammation. J. Leukoc. Biol. 74, 295–301. doi: 10.1189/jlb.1202628, PMID: 12885947

[ref322] XausJ.CardóM.ValledorA. F.SolerC.LloberasJ.CeladaA. (1999). Interferon γ induces the expression of p21waf-1 and arrests macrophage cell cycle, preventing induction of apoptosis. Immunity 11, 103–113. doi: 10.1016/S1074-7613(00)80085-0, PMID: 10435583

[ref323] XieX.LiF.ChenJ.-W.WangJ. (2014). Risk of tuberculosis infection in anti-TNF-α biological therapy: from bench to bedside. J. Microbiol. Immunol. Infect. 47, 268–274. doi: 10.1016/j.jmii.2013.03.005, PMID: 23727394

[ref324] XinP.XuX.DengC.LiuS.WangY.ZhouX.. (2020). The role of JAK/STAT signaling pathway and its inhibitors in diseases. Int. Immunopharmacol. 80:106210. doi: 10.1016/j.intimp.2020.10621031972425

[ref325] XiongW.WenQ.DuX.WangJ.HeW.WangR.. (2018). Novel function of cyclooxygenase-2: suppressing mycobacteria by promoting autophagy *via* the protein kinase B/mammalian target of rapamycin pathway. J. Infect. Dis. 217, 1267–1279. doi: 10.1093/infdis/jiy033, PMID: 29373690

[ref326] XuD.LiY.LiX.WeiL.-L.PanZ.JiangT.-T.. (2015). Serum protein S100A9, SOD3, and MMP9 as new diagnostic biomarkers for pulmonary tuberculosis by iTRAQ-coupled two-dimensional LC-MS/MS. Proteomics 15, 58–67. doi: 10.1002/pmic.201400366, PMID: 25332062

[ref327] YangD.FuX.HeS.NingX.LingM. (2017). Analysis of differentially expressed proteins in *Mycobacterium avium*-infected macrophages comparing with *Mycobacterium tuberculosis*-infected macrophages. Biomed. Res. Int. 2017:5103803. doi: 10.1155/2017/5103803, PMID: 28573139PMC5442340

[ref328] YangH.WangY.ZhangZ.LiH. (2020). Identification of KIF18B as a hub candidate gene in the metastasis of clear cell renal cell carcinoma by weighted gene co-expression network analysis. Front. Genet. 11:905. doi: 10.3389/fgene.2020.00905, PMID: 32973873PMC7468490

[ref329] YaoK.ChenQ.WuY.LiuF.ChenX.ZhangY. (2017). Unphosphorylated STAT1 represses apoptosis in macrophages during mycobacterium tuberculosis infection. J. Cell Sci. 130, 1740–1751. doi: 10.1242/jcs.200659, PMID: 28348106

[ref330] YarilinaA.Park-MinK.-H.AntonivT.HuX.IvashkivL. B. (2008). TNF activates an IRF1-dependent autocrine loop leading to sustained expression of chemokines and STAT1-dependent type I interferon–response genes. Nat. Immunol. 9, 378–387. doi: 10.1038/ni1576, PMID: 18345002

[ref331] YiF.HuJ.ZhuX.WangY.YuQ.DengJ.. (2021). Transcriptional profiling of human peripheral blood mononuclear cells stimulated by *Mycobacterium tuberculosis* PPE57 identifies characteristic genes associated with type I interferon signaling. Front. Cell. Infect. Microbiol. 11:716809. doi: 10.3389/fcimb.2021.716809, PMID: 34490145PMC8416891

[ref332] YuJ. S. L.CuiW. (2016). Proliferation, survival and metabolism: the role of PI3K/AKT/mTOR signalling in pluripotency and cell fate determination. Development 143, 3050–3060. doi: 10.1242/dev.137075, PMID: 27578176

[ref333] ZhangB.HorvathS. (2005). A general framework for weighted gene co-expression network analysis. Stat. Appl. Genet. Mol. Biol. 4:Article17. doi: 10.2202/1544-6115.1128, PMID: 16646834

[ref334] ZhangX.HuangT.WuY.PengW.XieH.PanM.. (2017). Inhibition of the PI3K-Akt-mTOR signaling pathway in T lymphocytes in patients with active tuberculosis. Int. J. Infect. Dis. 59, 110–117. doi: 10.1016/j.ijid.2017.04.004, PMID: 28416440

[ref335] ZhangT.RaoG.GaoX. (2021). Identification of hub genes in tuberculosis *via* bioinformatics analysis. Comput. Math. Methods Med. 2021:8159879. doi: 10.1155/2021/8159879, PMID: 34671419PMC8523273

[ref336] ZhangY.ZhangX.ZhaoZ.ZhengY.XiaoZ.LiF. (2019). Integrated bioinformatics analysis and validation revealed potential immune-regulatory miR-892b, miR-199b-5p and miR-582–5p as diagnostic biomarkers in active tuberculosis. Microb. Pathog. 134:103563. doi: 10.1016/j.micpath.2019.103563, PMID: 31175974

[ref337] ZhaoJ.GaoS.ChenC.LiH.WangS.YuY.. (2022). Screening and identification of differentially expressed long non-coding RNAs in multidrug-resistant tuberculosis. PeerJ 10:e12776. doi: 10.7717/peerj.12776, PMID: 35111403PMC8772445

[ref338] ZhouY.ShahS. Z. A.YangL.ZhangZ.ZhouX.ZhaoD. (2016). Virulent *Mycobacterium bovis* Beijing strain activates the NLRP7 inflammasome in THP-1 macrophages. PLoS One 11:e0152853. doi: 10.1371/journal.pone.0152853, PMID: 27043315PMC4820140

[ref339] ZitvogelL.KeppO.GalluzziL.KroemerG. (2012). Inflammasomes in carcinogenesis and anticancer immune responses. Nat. Immunol. 13, 343–351. doi: 10.1038/ni.2224, PMID: 22430787

